The article "Boosting Slime Mould Algorithm for High-Dimensional Gene Data Mining: Diversity Analysis and Feature Selection" was published in 2022. Journal: Comput Math Methods Med.

# Boosting Slime Mould Algorithm for High-Dimensional Gene Data Mining: Diversity Analysis and Feature Selection

**DOI:** 10.1155/2022/8011003

**Published:** 2022-10-13

**Authors:** Feng Qiu, Ran Guo, Huiling Chen, Guoxi Liang

**Affiliations:** ^1^Department of Computer Science and Artificial Intelligence, Wenzhou University, Wenzhou 325035, China; ^2^Cyberspace Institute Advanced Technology, Guangzhou University, Guangzhou 510006, China; ^3^Department of Information Technology, Wenzhou Polytechnic, Wenzhou 325035, China

## Abstract

Slime mould algorithm (SMA) is a new metaheuristic algorithm, which simulates the behavior and morphology changes of slime mould during foraging. The slime mould algorithm has good performance; however, the basic version of SMA still has some problems. When faced with some complex problems, it may fall into local optimum and cannot find the optimal solution. Aiming at this problem, an improved SMA is proposed to alleviate the disadvantages of SMA. Based on the original SMA, Gaussian mutation and Levy flight are introduced to improve the global search performance of the SMA. Adding Gaussian mutation to SMA can improve the diversity of the population, and Levy flight can alleviate the local optimum of SMA, so that the algorithm can find the optimal solution as soon as possible. In order to verify the effectiveness of the proposed algorithm, a continuous version of the proposed algorithm, GLSMA, is tested on 33 classical continuous optimization problems. Then, on 14 high-dimensional gene datasets, the effectiveness of the proposed discrete version, namely, BGLSMA, is verified by comparing with other feature selection algorithm. Experimental results reveal that the performance of the continuous version of the algorithm is better than the original algorithm, and the defects of the original algorithm are alleviated. Besides, the discrete version of the algorithm has a higher classification accuracy when fewer features are selected. This proves that the improved algorithm has practical value in high-dimensional gene feature selection.

## 1. Introduction

With the development of modern social science and technology, a variety of problems have arisen in the society, requiring researchers to design more efficient and novel methods to put forward feasible solutions. In recent years, some metaheuristic algorithms have been developed to solve various optimization problems. Some studies also show that metaheuristic methods are more effective than traditional gradient-based methods [1]. Metaheuristic algorithms can be divided into several categories according to their causes: evolutionary algorithm (EAs), such as genetic algorithm (GA) [2] and differential evolution (DE) [3], and swarm intelligence algorithms (SI), such as particle swarm optimization (PSO) [4], Harris hawks algorithm (HHO) [5], RUNge Kutta optimizer (RUN) [6], hunger games search (HGS) [7], slime mould algorithm (SMA) [8], monarch butterfly optimization (MBO) [9], moth search algorithm (MSA) [10], colony predation algorithm (CPA) [11], and weighted mean of vectors (INFO) [12]. In addition, they have been widely used in various fields, such as solar cell parameter Identification [13], economic emission dispatch problem [14], image segmentation [15, 16], plant disease recognition [17], medical diagnosis [18, 19], scheduling problems [20–22], optimization of machine learning model [23], multiobjective problem [24, 25], fault diagnosis [26], object tracking [27, 28], expensive optimization problems [29, 30], medical diagnosis [31, 32], combination optimization problems [33], feature selection [34, 35], practical engineering problems [36, 37], and robust optimization [38, 39].

The article "Boosting Slime Mould Algorithm for High-Dimensional Gene Data Mining: Diversity Analysis and Feature Selection" was published in 2022. Journal: Comput Math Methods Med.

Among all the algorithms, SMA is a new one proposed in recent years. Because of its excellent performance in dealing with complex problems and simple implementation, SMA has been widely applied in recent years. Because of its exploration and exploitation capabilities, it has been widely used in various fields to solve specific practical problems. For example, Kouadri et al. [40] proposed to use SMA in the actual power system to solve the optimal power problem and minimize the total cost of conventional and random power generation under the constraints of the power system. Khunkitti et al. [41] proposed the multiobjective optimal power flow (MOOPF) problem based on SMA, taking cost emission and transmission line loss as part of the objective function of the power system. Simulation results show that SMA has better solutions than other algorithms in the literature. Jafari-Asl et al. [42] proposed a method combining LS (line sampling) method with slime mould algorithm to solve the reliability problem under highly nonlinear and implicit limit states. Izci and Ekinci [43] evaluated the optimization ability of SMA by using a proportional integral derivative (PID) controller to adjust the speed of dc motor and maintain the terminal output of automatic voltage regulator (AVR) system and compared the performance of SMA with that of other controllers designed by competitive algorithms. Houssein et al. [44] proposed a multiobjective optimization algorithm based on SMA. The reliability of the proposed MOSMA was verified by the actual multiobjective optimization of automotive helical springs, and the effectiveness of MOSMA was evaluated by the Wilcoxon test and performance indicators. Houssein et al. [45] proposed a method combining SMA with adaptive guided differential evolution algorithm (AGDE) (SM-AGDE) to solve some of the defects of SMA. Gupta et al. [46] proposed a SMA to solve the estimation problem of proton exchange membrane fuel cell (PEMFC) model, which showed good performance in jumping out of local optimum, and the predicted results were basically consistent with the actual results. Therefore, SMA can be used for fuel cell problems. Elsayed et al. [47] used SMA to identify the parameters of transformer equivalent circuit and verified the ability and accuracy of SMA in parameter estimation of single-three-phase transformer, as well as its high performance and stability in determining the optimal parameters.

The article "Boosting Slime Mould Algorithm for High-Dimensional Gene Data Mining: Diversity Analysis and Feature Selection" was published in 2022. Journal: Comput Math Methods Med.

Hassan et al. [48] proposed an improved SMA (ISMA) to solve the problem of target and dual target economy and emission scheduling (EED) considering the valve point effect, in which the best solution was obtained by updating the position of the solution by using two equations in the sine and cosine algorithm. At the same time, on the basis of Pareto dominance concept and fuzzy decision, multiobjective ISMA is proposed, which has good performance and robustness. Jia et al. [49] optimized the SMA by introducing compound mutation strategy (CMS) and restart strategy (RS). CMS was used to increase population diversity, RS was used to avoid local optimization, and the effectiveness of the proposed CMSRSSMA was tested on the benchmark function. Meanwhile, the CMSRSSMA_SVM model was proposed and used for feature selection and parameter optimization. Altay [50] utilized 10 different chaotic mappings to generate chaotic rather than random values in SMA. By using chaotic mapping, the global convergence rate of SMA is improved and the local solution is avoided. Abdel-Basset et al. [51] integrated SMA and WOA algorithms to maximize Kapur's entropy and applied them in the field of image segmentation, achieving good results. Chauhan et al. [52] proposed a method combining arithmetic optimizer algorithm (AOA) and slime mould algorithm (SMA), namely, HAOASMA algorithm, which solved the problems of slime mould algorithm's insufficient memory and slow local convergence speed.

Since SMA was proposed, it has been applied in various fields and used to solve various problems, showing good performance. However, in the face of some complex optimization tasks, there are still problems of falling into local optimum and slow convergence. In order to cope with this situation and improve the performance of the algorithm, a combinatorial optimization method (GLSMA) based on Gaussian mutation and Levy flight is proposed in this paper. In GLSMA, the global exploration and local exploitation capabilities of the original algorithm are improved by introducing Gaussian mutation and Levy flight mechanism. In the optimization iteration process, the original position of slime moulds in the population was modified by Gaussian to enhance the diversity of the population and improve the global exploration ability of the algorithm, so that the algorithm could achieve a balance between global exploration and local exploitation. After that, Levy flight was used to improve the randomness of SMA and to jump out of local optimum. Benchmark function test results show that the improved version of GLSMA has better global search and local exploration ability compared with other advanced algorithms. The discrete version based on GLSMA also shows an ideal effect on feature selection.

The article "Boosting Slime Mould Algorithm for High-Dimensional Gene Data Mining: Diversity Analysis and Feature Selection" was published in 2022. Journal: Comput Math Methods Med.

The contributions and highlights of this paper are summarized below:

1. An improved slime mould algorithm (GLSMA) based on Gaussian mutation and Levy flight is proposed to solve continuous optimization problems and high-dimensional gene feature selection problems
2. The superiority of GLSMA is proved by comparing with several well-known algorithms on public datasets and achieved good results
3. Proposed binary GLSMA to solve high-dimensional gene feature selection problems
4. The developed GLSMA has faster exploration speed and convergence speed in the global optimization task
5. Binary GLSMA has the highest classification accuracy and the least number of features in high-dimensional gene feature selection task

The remainder of this paper is organized as follows: the second part introduces the original SMA. The third part introduces Gaussian mutation mechanism and Levy flight in detail, as well as the improved SMA based on the two mechanisms. The fourth part introduces a series of comparison experiments between GLSMA and other similar algorithms, including comparison experiments on continuous function and discrete function. The fifth part reviews and discusses of the proposed work. The sixth part summarizes the conclusions of this paper and gives several directions of future work.

## 2. Slime Mould Algorithm

Li et al. [8] established a mathematical model based on the oscillation behavior of slime moulds and thus proposed a metaheuristic slime mould algorithm (SMA).

The mathematical formula of slime moulds is shown in

(1) $$\begin{array}{c} X\left(t+1\right)=\left\{\begin{array}{c} \mathrm{rand}∙\left(\text{UB}-\text{LB}\right)+\text{LB},\;\mathrm{rand}<z,\\ X_{b}\left(t\right)+\text{vb}\left(t\right)∙\left(W∙X_{A}\left(t\right)-X_{B}\left(t\right)\right),r<p,\\ \text{vc}\left(t\right)∙X\left(t\right),r\geq p, \end{array}\right. \end{array}$$

where vb represents a random value in the interval [−*a*, *a*]. Parameter vc ranges in the interval [−*b*, *b*], which decreases with the number of iterations. Through the cooperative interaction between vb and vc, the selection behavior of slime moulds can be simulated and the optimal solution can be selected. *Max*_*t*_ indicates the maximum number of iterations. UB and LB represent the upper and lower boundaries of the search space, respectively. *X*_*b*_ represents the position vector of the current highest fitness (highest concentration) individual. *X*_*A*_(*t*) and *X*_*B*_(*t*) represent the position vectors of random individuals selected from the slime moulds in the *t* iteration. rand and *r* are the random values between 0 and 1. Parameter *z* is set to 0.03. *X*(*t*) and *X*(*t* + 1) represent position vectors of slime moulds at the *t* and (*t* + 1) iterations, respectively.

(2) $$\begin{array}{c} a=\mathrm{arctanh}\left(1-\left(\frac{t}{{\mathrm{Max}}_{t}}\right)\right), \end{array}$$

(3) $$\begin{array}{c} b=1-\left(\frac{t}{\text{Ma}{\text{x}}_{t}}\right). \end{array}$$

In addition, the decision parameter *p* can be calculated as follows:

(4) $$\begin{array}{c} p=\tanh\left|S\left(i\right)-\text{DF}\right|, \end{array}$$

where *S*(*i*) indicates the fitness of the ith individual in the slime mould, *i* ∈ 1, 2, ⋯, *N*; *N* denotes the size of population; and DF represents the best fitness, which is attained during all of the iterations.

(5) $$\begin{array}{c} W\left(\text{SmellIndex}\left(i\right)\right)=\left\{\begin{array}{c} 1+r∙\log\left(\frac{\text{bF}-\text{SmellOrder}\left(i\right)}{\text{bF}-\text{wF}}+1\right),\text{condition},\\ 1-r∙\log\left(\frac{\text{bF}-\text{SmellOrder}\left(i\right)}{\text{bF}-\text{wF}}+1\right),\text{otherwise}, \end{array}\right.\; \end{array}$$

(6) $$\begin{array}{c} \left[\text{SmellOrder},\text{SmellIndex}\right]=\text{sort}\left(S\right), \end{array}$$

where *W*  is the weight vector of slime moulds and *bF* and *wF* are the best and worst fitness obtained in the current iteration, respectively. SmellIndex and SmellOrder represent fitness ordering order (minimum problems are sorted in ascending order) and corresponding fitness values, respectively. condition represents the first half of SmellOrder.

The article "Boosting Slime Mould Algorithm for High-Dimensional Gene Data Mining: Diversity Analysis and Feature Selection" was published in 2022. Journal: Comput Math Methods Med.

## 3. Description of the GLSMA

### 3.1. Gaussian Mutation

Gaussian mutation (GM) operator is derived from Gaussian normal distribution, which is distinguished from Cauchy distribution. In the vertical direction, the Gaussian distribution is larger than the Cauchy distribution, and in the horizontal direction, the Gaussian distribution is smaller than the Cauchy distribution. Gauss mutations are more likely to produce new offspring in this part because of their narrow tail. In response, the search equation takes smaller steps to explore every corner of the search space in a better way. The Gaussian density function can be described as

(7) $$\begin{array}{c} f_{\text{Gaussian}\left(0,\sigma^{2}\right)}\left(\propto \right)=\frac{1}{\sqrt{2\pi \sigma^{2}}}e^{-\sigma^{2}/2\sigma^{2}}, \end{array}$$

where *σ*^2^ is the variance of each member of the population. By setting the mean to 0 and the standard deviation to 1, this function is further simplified to generate an *N*-dimensional random variable. The generated random variables were applied to the exploration stage of slime moulds, as shown below:

(8) $$\begin{array}{c} X_{i}^{\prime }=X_{i}\times \left(1+G\left(\propto \right)\right), \end{array}$$

where *G*(∝) is a uniformly distributed random number derived from Gaussian distribution, *X*_*i*_  is a position in SMA during the current iteration, and *X*_*i*_′ is the position corresponding to *X*_*i*_ after Gaussian mutation. The introduction of Gaussian mutation mechanism enhances the diversity of population and improves the quality of SMA solution.

### 3.2. Levy Flight

Levy flight (LF) was first proposed by French mathematician Paul Levy in 1937, after which researchers used Levy statistics to describe various natural phenomena. Levy flight operator improves slime mould search capability by helping all search agents advance to better, more promising positions. A simple description of the Levy distribution is as follows:

(9) $$\begin{array}{c} \text{Levy}\left(\beta \right)\sim u=t^{-1-\beta },0<\beta \leq 2, \end{array}$$

where *β* is an important index of regulatory stability. Levy random numbers can be described by the following formula:

(10) $$\begin{array}{c} \text{Levy}\left(\beta \right)\sim \frac{\varphi \times \mu }{{\left|v\right|}^{1/\beta }}, \end{array}$$

where *μ* and *v*  are standard normal distributions, Γ is a standard gamma function, *β* is set to 1.5, and *φ* is defined as follows:

(11) $$\begin{array}{c} \varphi ={\left[\frac{\Gamma \left(1+\beta \right)\times \sin\left(\pi \times \beta /2\right)}{\Gamma \left(\left(\left(1+\beta \right)/2\right)\times \beta \times 2^{\left(\beta -1\right)/2}\right)}\right]}^{1/\beta }. \end{array}$$

In the exploration phase of slime mould algorithm, Levy strategy was used to update the location of search agents, so as to better balance exploration and search capabilities. The update formula is as follows:

(12) $$\begin{array}{c} X_{i}^{\prime }=X_{i}\times \left(1+\text{Levy}\left(\beta \right)\right). \end{array}$$

In the formula, Levy(*β*) is taken from the Levy distribution and is the number of random distribution. *X*_*i*_′ is the new location of the *i*-th search agent *X*_*i*_ after the update. The introduction of Levy flight can help all individuals to jump out of local optimum and improve the quality of the population.

The article "Boosting Slime Mould Algorithm for High-Dimensional Gene Data Mining: Diversity Analysis and Feature Selection" was published in 2022. Journal: Comput Math Methods Med.

### 3.3. Framework of Proposed GLSMA

In this section, we will describe GLSMA based on the Gaussian mutation mechanism and Levy flight strategy in detail. In the process of algorithm improvement, adding a mechanism can generally improve the algorithm in only one aspect but cannot improve the global exploration and local exploitation ability at the same time. By adding the Gaussian mutation mechanism, the corresponding value can be obtained from the current solution, but this can only improve the local exploitation ability and will fall into local optimal. The Levy flight mechanism can expand the search range of solutions, increase the possibility of obtaining the optimal solution, and avoid falling into local optimal. As a result, in the original SMA, two strategies (GM and LF) were introduced to facilitate the coordination of global exploration and local exploitation, forming a new SMA variant.

In the process of iterative optimization, Gaussian mutation was considered for individuals in the slime mould individuals after initial updating. The individuals obtained after mutation were compared with the individuals without that. If the fitness of the individuals in the mutation state was not improved, the original individuals were retained and the mutant individuals were discarded to ensure the quality of the population. Considering that the algorithm is easy to fall into local optimum, levy flight strategy is introduced to improve the randomness of SMA and the ability of jumping out of local optimum. The flowchart of GLSMA is shown in Figure 1. Experimental results show that compared with other swarm intelligence algorithms, GLSMA not only has stronger global exploration ability but also contributes to increase the quality of solutions and speed up convergence. The structure of the proposed GLSMA optimizer is shown in Algorithm 1.

### 3.4. Computational Complexity Analysis

According to the structure of GLSMA, it mainly includes initialization, fitness evaluation, fitness ranking, weight updating, position updating based on SMA strategy, position adjustment based on Gaussian mutation mechanism, and position updating based on Levy flight strategy, where *N* is the number of slime moulds, *D* is the function's dimension, and *T* is the maximum number of iterations. The calculation is as follows:

The time complexity for initialization is *O*(*D*). In evaluating and ordering fitness, the computational complexity is *O* (*N* + *N* log*N*). The computational complexity of the update weight is *O*(*N* × *D*). The computational complexity of position updating process based on SMA is *O*(*N* × *D*). Similarly, the computational complexity of position updating process based on Gaussian mutation mechanism is *O*(*N* × *D*). The computational complexity of the position update process based on Levy flight is *O*(*N* log*D*). Therefore, the total computational complexity of GLSMA is *O*(*D* + *T* × *N* × (1 + 3*D* + log*D* + log*N*)).

The article "Boosting Slime Mould Algorithm for High-Dimensional Gene Data Mining: Diversity Analysis and Feature Selection" was published in 2022. Journal: Comput Math Methods Med.

## 4. Experiments and Results

In the experiment, to evaluate the continuous and discrete versions of GLSMA, the proposed SMA algorithm is compared with other optimizers on the continuous functions and feature problems, respectively. The effectiveness and competitiveness of the proposed algorithm are verified by two parts of experiments. In the first part, the strategies added on SMA were tested on 23 benchmark test functions (including 7 unimodal functions, 6 multimodal functions, and more than 10 fixed dimension multimodal functions) and 10 classic CEC2014 benchmark test functions (including 2 hybrid functions and 8 composition functions), to see whether the mechanism has a positive effect on the algorithm. Then, in the same test environment, GLSMA is compared with some original algorithms and advanced MA algorithms. In the second part, we compare the proposed binary GLSMA (BGLSMA) with other classifiers on feature selection problems.

All GLSMA experiments were written in the MATLAB R2014a compiler and run on Windows 10(64-bit) operating system. The computer hardware is Intel(R) Xeon(R) Silver 4110 CPU (2.40 GHz) 2.10 GHz (dual processors) and 32GB RAM.

In Section 4.1, we will test the influence of different mechanisms on the algorithm. In Section 4.2, GLSMA is compared with seven metaheuristic algorithms to prove its effectiveness. In Section 4.3, GLSMA is compared with eight advanced algorithms to verify its ability on exploration and exploitation. In Section 4.4, we use binary GLSMA (BGLSMA) to deal with feature selection in 14 UCI datasets.

### 4.1. The Influence of Gaussian Mutation and Levy Flight

As mentioned above, GLSMA consists of two main improved strategies: Gaussian mutation mechanism and Levy flight strategy. The purpose of this section is to validate the effectiveness of the combination of the two strategies. To this end, we compare GLSMA, SMA, and their variants GSMA and LSMA on 33 benchmark functions. GSMA only uses Gaussian mutation strategy, LSMA only uses Levy flight strategy, and SMA is the original algorithm.

All algorithm tests were carried out under the expected conditions to eliminate the influence of irrelevant factors on the experiment and ensure the fairness of the test. The population size was set to 30; the maximum evaluation test was uniformly set to 300,000. In order to weaken the influence of algorithm randomness on the experiment, we conducted 30 independence tests for each test case. In this paper, the average value of optimal function (Avg) and standard deviation (Std) of the selection algorithm results are compared. The global exploration ability and result quality of the algorithm were evaluated on the average (Avg), and Std of the optimal function was used to evaluate the robustness of the algorithm. In order to show the best results more clearly, all the best results are italicized.

The article "Boosting Slime Mould Algorithm for High-Dimensional Gene Data Mining: Diversity Analysis and Feature Selection" was published in 2022. Journal: Comput Math Methods Med.

In addition, nonparametric statistical verification Wilcoxon signed-rank test was used to measure the degree of improvement and whether it was statistically significant. The significance level was set at 0.05. The symbolic label “+/=/-” in the results states that the proposed method GLSMA is superior to, equal to, and inferior to other methods of competition, respectively. For a comprehensive statistical comparison, the Friedman [53] test was used to evaluate the average behavior of all different algorithms for further statistical comparison, and the average ranking was given in these comparison results, and the average rank value (ARV) of the Friedman test was used to evaluate the average performance of the compared methods.

Tables 1–4 contain 23 benchmark functions and 10 test functions in CEC2014. The selected 33 test functions include several different problems, covering unimodal function, multimodal function, fixed dimension multimodal function, hybrid function, and composition function. These test functions can be used to test the algorithm's global exploration capabilities and local exploitation capabilities and can be used to verify the balance between exploration and exploitation capabilities.

As can be seen from the results in Tables 5 and 6, GLSMA is significantly superior to other mechanism combinations and the original SMA. After careful analysis, Avg and Std in Table 5 represent the superiority of GLSMA over F1-F7, F9-F14, F17-F18, and F22-F33 functions. On the test functions F1-F4, F9-F11, F26-F28, and F30-F33, the GLSMA's Std value is 0, indicating that GLSMA has strong robustness. This is because the combination of Gaussian mutation and Levy flight mechanism improves the performance of the original SMA and can successfully find global optimal solutions for various complex problems. According to the statistical results of *p* value in Table 6, many values of SMA column are less than 0.05, indicating that GLSMA has a certain improvement on the original SMA. As can be seen from the ARV tested by Friedman in Table 7, when comparing the four algorithms, GLSMA ranks first and is significantly superior to other algorithms. Moreover, it can be seen that the improvement effect of Gaussian mutation mechanism or Levy flight mechanism on the original SMA is not good, even can be said to be poor, but the combination of the two can achieve a good balance between exploration and exploitation, so as to achieve a good effect. In summary, the results show that the addition of Gaussian mutation mechanism and Levy flight mechanism is not only beneficial to the exploration and exploitation ability of GLSMA but also beneficial to the balance between the exploitation and exploration ability of GLSMA, which has a certain positive effect on the algorithm and improves the robustness of the original algorithm, which has improved significance.

The article "Boosting Slime Mould Algorithm for High-Dimensional Gene Data Mining: Diversity Analysis and Feature Selection" was published in 2022. Journal: Comput Math Methods Med.

Compared with the table, the image can more intuitively and clearly reflect the optimization results of GLSMA compared with other comparison objects.  Figure 2 shows the convergence curves of the four comparison methods on nine functions. It is obvious that GLSMA using two mechanisms achieves better results than its variants. The combination of Gaussian mutation and Levy flight enables GLSMA to escape from local traps faster and obtain the global optimal solution. In the meantime, it can be seen that GLSMA has the fastest rate of convergence and can get the optimal value first. The results show that this combination of mechanisms can quicken the convergence of the algorithm while jumping out of local optimum. In general, the combination of GM and LF improves the overall performance of the original SMA.

### 4.2. Comparison with Well-Known Algorithms

In this experiment, 23 classical functions and 10 of the CEC2014 benchmark functions were selected to evaluate the performance of GLSMA. The 33 benchmark test functions used in all experiments of continuous optimization can be divided into four categories: unimodal function, multimodal function, hybrid function, and composition function. The unimodal function (F1-F7) has only one solution, which can be used to test the development ability of the algorithm. The multimodal function (F8-F23) has several local optimal solutions and is suitable for verifying the exploration ability of the algorithm. The hybrid function and composition function (F24-F33) selected from CEC2014 are used to verify the balance between algorithm exploration and exploitation. These functions are often used to assess the overall power of algorithms. In this experiment, the performance of the improved GLSMA was compared with PSO [4], WOA [54], GWO [55], SCA [56], FOA [57], DE [3], and SSA [58].

The article "Boosting Slime Mould Algorithm for High-Dimensional Gene Data Mining: Diversity Analysis and Feature Selection" was published in 2022. Journal: Comput Math Methods Med.

Tables 8–10 record the comparison results of GLSMA with seven well-known algorithms. The comparison results are shown in Table 10; among GLSMA and seven famous algorithms, the average Friedman test result of GLSMA is 2.328283, ranking first, and the average Friedman test result of DE is 2.730303, ranking second. It is obvious that the Friedman test of GLSMA and DE is obviously better than other algorithms. The average value (Avg) and standard deviation (Std) of optimal solution of GLSMA and other well-known algorithms are shown in Table 8. GLSMA has a significant advantage. Moreover, in all the comparison algorithms, GLSMA has Std 0 on more test functions, which proves that GLSMA algorithm has stronger stability. In addition, GLSMA shows obvious advantages and stability in almost all of the composition functions (F26-F28 and F30-F33).  Table 9 shows the Wilcoxon symbol test results between GLSMA and other well-known algorithms. It can be seen that the *p* value of GLSMA is less than 0.05 on almost all benchmark functions, which proves that GLSMA is significantly better than other algorithms, especially FOA, in all functions. Therefore, compared with these basic metaheuristic algorithms, GLSMA has statistical significance.

From the convergence curves of 8 algorithms on 9 functions shown in Figure 3, it can be seen that GLSMA improves the global search ability under the dual mechanism and can quickly escape from the local optimal trap and faster to find the global optimal.

In conclusion, compared with other well-known algorithms, GLSMA shows good overall superiority and stability. The strategy combination of Gaussian mutation and Levy flight enables the proposed GLSMA to obtain higher quality solutions in the optimization process, thus achieving a balance between exploration and exploitation.

### 4.3. Comparison with Advanced Algorithms

In this experiment, the proposed GLSMA algorithm is compared with 8 classical advanced algorithms in order to fully prove its global search and avoiding local optimality, including MPEDE [59], LSHADE [60], ALCPSO [61], CLPSO [62], CMAES [63], BMWOA [64], CESCA [65], and IGWO [66]. These include two classic DE variants, two superior PSO variants, and variations of WOA and GWO algorithms.

The comparison results of GLSMA with eight advanced algorithms are shown in Tables 11–13.  Table 11 shows the average value and standard deviation of the optimal solution obtained by GLSMA and advanced algorithms. As can be seen, compared to other algorithms, GLSMA shows good superiority and stability in F1-F5, F7-F11, F13, F15, F21, F26-F28, and F30-33 functions.  Table 12 shows the Wilcoxon rank test result's *p* value among GLSMA and eight advanced algorithms. From the table values, it can be seen that GLSMA outperforms other comparison algorithms on most benchmark functions. GLSMA is superior to CESCA in all functions. Therefore, GLSMA is obviously competitive with other excellent algorithms.  Table 13 shows the comparison results; among GLSMA and other 8 advanced algorithms, the average Friedman test result of GLSMA ranks the first, which is 3.629293.

The article "Boosting Slime Mould Algorithm for High-Dimensional Gene Data Mining: Diversity Analysis and Feature Selection" was published in 2022. Journal: Comput Math Methods Med.

The convergence curves of all nine algorithms on nine functions shown in Figure 4 show that GLSMA's convergence speed is faster than other advanced algorithms, and it can jump out of local optimum faster and avoid falling into local optimum better than other algorithms.

In summary, the introduction of Gaussian mutation mechanism and Levy flight mechanism gives GLSMA an advantage over competitive advanced algorithms, showing superior performance in different types of functions. GLSMA not only has stronger global search ability but also can avoid falling into local optimum.

### 4.4. The Experiments for Feature Selection

In this section, we transform the proposed algorithm GLSMA into a discrete version, namely, BGLSMA, which is applied to feature selection problems of high-dimensional gene data, thus making the proposed algorithm more realistic.

The purpose of feature selection problem is to remove some redundant and irrelevant features from the sample, so as to reduce the complexity of feature selection problem, reduce the subsequent calculation cost, and obtain higher classification accuracy. In the process of feature selection, it is necessary to determine which features should be selected. As a result, we transform continuous GLSMA into discrete GLSMA, namely, BGLSMA. The proposed GLSMA increases the population diversity, strengths the local exploitation ability, and helps us select favorable features in the search space, so as to obtain better feature subsets and improve classification accuracy.

#### 4.4.1. Binary GLSMA

In feature selection algorithm based on GLSMA, *x* = (*x*_*i*,1_, *x*_*i*,2_, ⋯, *x*_*i*,*n*_) represents a subset of features. In BGLSMA, if *x*_*i*,1_ = 1, this feature is selected, and conversely, if *x*_*i*,1_ = 0, this feature is discarded. In order to solve discretization problems, GLSMA needs to be discretized. The individual with binary position vector is initialized by random threshold, and then, the discretization of position *X*_*i*_ can be expressed as

(13) $$\begin{array}{c} X_{i}^{j}\left(t+1\right)=\left\{\begin{array}{c} 1,\text{if}\mathrm{rand}\geq T\left(X_{i}^{j}\left(t\right)\right),\\ 0,\text{if}\mathrm{rand}<T\left(X_{i}^{j}\left(t\right)\right), \end{array}\right.\\ T\left(x\right)=\frac{1}{1+e^{-2x}} \end{array}$$

In the formula above, *X*_*i*_(*t* + 1) indicates the value of the *i*-th dimension of the agent individual position *X* searched in the discrete space, and rand means a random number within the range of [0, 1]. *T*(*x*) means converting the value of the *i*-th dimension of *X* in the continuous motion space to 0 or 1, thus realizing the discretization of the continuous space. The transformation of *T*(*x*) does not change the structure of the algorithm.

The article "Boosting Slime Mould Algorithm for High-Dimensional Gene Data Mining: Diversity Analysis and Feature Selection" was published in 2022. Journal: Comput Math Methods Med.

As described above, feature selection is a process of using the least gene subset to obtain the optimal classification accuracy, that is, to improve the classification accuracy and reduce the number of features. This problem is described as a combinatorial optimization problem. In order to satisfy each objective, a linear combination of feature number and error rate is used to define fitness function, and the candidate solutions are evaluated comprehensively.

(14) $$\begin{array}{c} \text{ fit}=\alpha \cdot E+\beta \cdot \frac{R}{D}. \end{array}$$

In the above formula, *E* is the classification accuracy rate of KNN classifier, the length of selected feature subset is represented by *R*, and the total number of features in the dataset is represented by *D*. *α* and *β* are the weights of classification error rate and feature reduction, respectively. Compared with feature reduction, more attention is paid to accuracy; we set *α* to 0.95 and the latter to 0.05.

#### 4.4.2. Simulation Experiments

In this experiment, the resulting BGLSMA is compared with other excellent metaheuristic optimizers on 14 UCI feature selection datasets. In Table 14, the details of these datasets are shown, including the number of samples, the number of features, and the number of categories. Table 14 shows that, in these datasets, the sample number is 50-308, the feature number is 2000-15010, and the number of categories is 2-11. These datasets contain several different types of data. These high-dimensional gene datasets have such characteristics: the sample number is small, and the feature number is thousands, which has some impact on data dimension reduction.

In order to select fewer features while maintaining classification accuracy, K-nearest neighbor (KNN) [67] algorithm is used for data classification. K-nearest neighbor is a nonparametric regression statistical method with wide application in classification problems. The steps of KNN algorithm are as follows: firstly, the original data is preprocessed, and the processed data is divided into training set and test set; second, set the appropriate parameter *k* to 1. Then, the initial group is selected in the training set, and the distance *D* between the initial group and the test group is calculated. The distance calculation formula is shown in Equation (15). At the same time, calculate the distance *L* between the training group and the test group, and compare whether *L* is less than *D*. If *L* is less than *D*_max_, repeat the above steps until the termination condition is reached.

(15) $$\begin{array}{c} D\left(x,y\right)={\left(\overset{N}{\underset{k}{\sum }}\left(x_{k}-y_{k}\right)\right)}^{1/2}. \end{array}$$

Metaheuristic classifiers used for comparison include bGWO [68], BBA [69], BGSA [70], BPSO [71], bALO [72], BSSA [73], and, the binary form of the original SMA, BSMA. The above classifiers are used for feature selection, and the relevant data of feature subsets found by various algorithms in the search process are learned in KNN classifier, and the corresponding result information is finally output for comparison. In order to reduce the influence of random factors, 10-fold cross validation was adopted, and the average value of multiple cross experimental results was taken as the result to evaluate the algorithm's accuracy.

The article "Boosting Slime Mould Algorithm for High-Dimensional Gene Data Mining: Diversity Analysis and Feature Selection" was published in 2022. Journal: Comput Math Methods Med.

Tables 15–18 list the statistical results of the average number of selected features, the average error rate, the average fitness, and the average calculation time. According to the average number of selected features in Table 15, the proposed BGLSMA has the least average number of selected features in all datasets except Tumors_11 and Tumors_14. On Colon and Leukemia datasets, BGLSMA obtained a small selected feature with a standard deviation less than 1. This proves that GLSMA can obtain fewer features and higher classification accuracy. As can be seen from the tables, BGLSMA has higher classification accuracy in processing some complex high-dimensional data and can find smaller number of features and reduce the data scale. In terms of ARV index, BGLSMA ranks first. This suggests that BGLSMA can obtain very competitive results in terms of the number of features selected.

Table 16 shows the comparison results of eight algorithms in terms of average error rate. It can be seen from the ranking that BGLSMA has the lowest average error rate, which proves that the proposed algorithm not only has better performance in global optimization problems but also has good classification ability in feature selection optimization. It can be seen that the average error rate of BGLSMA is significantly lower than that of BSMA. The Gaussian mutation mechanism enables the population to search a larger space. As the number of iterations increases, the most representative features in each dataset are gradually selected, and the classification accuracy is also improved.

The article "Boosting Slime Mould Algorithm for High-Dimensional Gene Data Mining: Diversity Analysis and Feature Selection" was published in 2022. Journal: Comput Math Methods Med.

It is clear from the key measurements listed in Table 17, namely, the weighted number of features and the weighted error rate, that BGLSMA outperformed other competitors on 78.6% of the dataset. In addition, both the detailed data and the final ARV value show that BGLSMA has greatly improved compared with BSMA, which is due to the introduction of Levy flight mechanism, which increases the diversity and randomness of the population and selects features from a wider range of features, thus achieving higher classification accuracy.

Table 18 shows the average calculation time results of algorithm comparison. The computation cost of BGLSMA optimizer proposed in this paper is higher than that of BBA, BGSA, and other optimizers, and the time complexity of the BSMA and bGWO with better performance is also higher than that of other optimizers, as shown in Tables 15–18. The introduction of GM and LF strategies not only improves the performance of BGLSMA but also increases the cost of computing time. Meanwhile, the time cost of the original SMA is higher than that of other algorithms, which leads to the high time cost of BGLSMA to a certain extent.

To sum up, BGLSMA is found to be the best optimizer in the overall comparison with other optimizers. Although the time cost is relatively high, BGLSMA can select the optimal feature subset on the vast majority of high-dimensional gene datasets without losing meaningful features and achieve the best fitness and classification error rate at the same time. The experimental results show that the combined strategy of Gaussian mutation and Levy flight guarantees the good results of GLSMA in global exploration.

## 5. Discussions

In this part, the GLSMA algorithm proposed in this paper, its advantages, and the points that can be improved are discussed. In the original SMA, the slime mould is not able to find the optimal solution in the search space, and it will fall into the local optimum when encountering some problems, which limits the use of the algorithm. In this paper, Gaussian mutation and Levy flight are introduced to update the population, which can enhance the global exploration ability and avoid the algorithm falling into local optimum. Experimental results show that the optimization effect of the dual mechanism is better than that of the single mechanism, and the optimization effect of GLSMA is better than some advanced optimization algorithms.

We monitor the situation after the population updates its optimal fitness value to determine whether it falls into local optimum. If it falls into local optimum, then Levy flight mechanism is invoked to help the algorithm increase the search space and jump out of local trap. The combination of the dual mechanism is significantly better than the single mechanism. However, it can be seen from Table 18 that the time cost of BGLSMA is relatively high, which is partly due to the high time cost of BSMA and partly due to the addition of mechanism, which leads to the increase of time cost. Correspondingly, the mechanism greatly improves the performance of the algorithm, allowing it to be applied to more domains, such as human activity recognition [74], microgrid planning [75], medical image augmentation [76], autism spectrum disorder classification [77], disease prediction [78, 79], named entity recognition [80], information retrieval services [81–83], and recommender systems [84–87].

The article "Boosting Slime Mould Algorithm for High-Dimensional Gene Data Mining: Diversity Analysis and Feature Selection" was published in 2022. Journal: Comput Math Methods Med.

## 6. Conclusions and Future Directions

In this paper, an improved SMA (GLSMA) algorithm based on Gaussian mutation and Levy flight is proposed. Experimental results show that the two mechanisms play an important role in further enhancing the global search of SMA and alleviating falling into local optimum. Firstly, the effectiveness of GLSMA method is verified by comparison with DE, PSO, GWO, and other well-known algorithms. Secondly, compared with other advanced swarm intelligence algorithms, such as MPEDE, LSHADE, ALCPSO, and CLPSO, GLSMA is able to find the optimal solution faster. Finally, in order to prove the performance of GLSMA in practical applications, BGLSMA is obtained by mapping GLSMA into binary space through transformation function, and it is applied to feature selection problems of 14 commonly used UCI high-dimensional gene datasets. Compared with excellent metaheuristic optimizer, general average characteristics selected number, average error rate, and average fitness and calculated the cost four aspects; it can be seen that GLSMA in the application of feature selection still has good global search ability and be able to select fewer features and higher classification accuracy. Therefore, the above conclusions indicate that GLSMA can be a promising method for not only function optimization problems but also practical feature selection problems.

There are still many aspects to explore in our research. We can consider applying GLSMA to other feature selection datasets and study the effectiveness of BGLSMA on other datasets. Further improvements to the SMA can be attempted to improve the balance between global exploration and local development. Finally, it is an interesting topic to apply SMA to more fields, such as photovoltaic parameter optimization and image segmentation (see Tables 5–18).

## Figures and Tables

**Figure 1:** Flowchart of the proposed GLSMA.

The article "Boosting Slime Mould Algorithm for High-Dimensional Gene Data Mining: Diversity Analysis and Feature Selection" was published in 2022. Journal: Comput Math Methods Med.

**Figure 2:** Convergence curves of GLSMA, SMA, GSMA, and LSMA on nine selected benchmark functions.

**Figure 3:** Convergence curves of GLSMA and seven original metaheuristic algorithms on nine selected benchmark functions.

**Figure 4:** Convergence curves of GLSMA and eight advanced algorithms on nine selected benchmark functions.

**Algorithm 1:** Pseudocode of GLSMA.

**Table 1:** Descriptions of unimodal benchmark functions.

Function	Dim	Range	*f*_min_
*F*_1_(*x*) = ∑_*i*=1_^*n*^*x*_*i*_^2^	30	[-100, 100]	0
*F*_2_(*x*) = ∑_*i*=1_^*n*^|*x*_*i*_| + ∏_*i*=1_^*n*^|*x*_*i*_|	30	[-10, 10]	0
*F*_3_(*x*) = ∑_*i*=1_^*n*^ (∑_*j*−1_^*i*^ *x*_*j*_)^2^	30	[-100, 100]	0
*F*_4_(*x*) = max_*i*_{|*x*_*i*_|, 1 ≤ *i* ≤ *n*}	30	[-100, 100]	0
*F*_5_(*x*) = ∑_*i*=1_^*n*−1^[100(*x*_*i*+1_ − *x*_*i*_^2^)^2^ + (*x*_*i*_ − 1)^2^]	30	[-30, 30]	0
*F*_6_(*x*) = ∑_*i*=1_^*n*^([*x*_*i*_ + 0.5])^2^	30	[-100, 100]	0
*F*_7_(*x*) = ∑_*i*=1_^*n*^*ix*_*i*_^4^ + random[0, 1]	30	[-128, 128]	0

**Table 2:** Descriptions of multimodal benchmark functions.

Function	Dim	Range	*f*_min_
$F_{8}\left(x\right)=\sum_{i=1}^{n}-x_{i}\sin\left(\sqrt{\left|x_{i}\right|}\right)$	30	[-500, 500]	−418.9829 × 30
*F*_9_(*x*) = ∑_*i*=1_^*n*^[*x*_*i*_^2^ − 10cos(2*πx*_*i*_) + 10]	30	[-5.12, 5.12]	0
$F_{10}\left(x\right)=-20\exp\left(-0.2\sqrt{1/n\sum_{i=1}^{n}x_{i}^{2}}\right)-\exp\left(1/n\sum_{i=1}^{n}\cos\left(2\pi x_{i}\right)\right)+20+e$	30	[-32, 32]	0
$F_{11}\left(x\right)=1/4000\sum_{i=1}^{n}x_{i}^{2}-\prod_{i=1}^{n}\cos\left(x_{i}/\sqrt{i}\right)+1$	30	[-600, 600]	0
$F_{12}\left(x\right)=\frac{\pi }{n}\left\{10\sin\left(\pi y_{1}\right)+\overset{n-1}{\underset{i=1}{\sum }}{\left(y_{i}-1\right)}^{2}\left[1+10\sin^{2}\left(\pi y_{i+1}\right)\right]+{\left(y_{n}-1\right)}^{2}\right\}+\overset{n}{\underset{i=1}{\sum }}u\left(x_{i},10,100,4\right)$ $y_{i}=1+\frac{x_{i}+1}{4}$ $u\left(x_{i},a,k,m\right)=\left\{\begin{array}{cc} k{\left(x_{i}-a\right)}^{m} & x_{i}>a\\ 0 & -a<x_{i}<a\\ k{\left(-x_{i}-a\right)}^{m} & x_{i}<-a \end{array}\right.$	30	[-50, 50]	0
*F*_13_(*x*) = 0.1{sin^2^(3*πx*_1_) + ∑_*i*=1_^*n*^(*x*_*i*_ − 1)^2^[1 + sin^2^(3*πx*_*i*_ + 1)] + (*x*_*n*_ − 1)^2^[1 + sin^2^(2*πx*_*n*_)]} + ∑_*i*=1_^*n*^*u*(*x*_*i*_, 5,100,4)	30	[-50, 50]	0

**Table 3:** Descriptions of fixed dimension multimodal benchmark functions.

Function	Dim	Range	*f*_min_
*F*_14_(*x*) = (1/500 + ∑_*j*=1_^25^(1/*j* + ∑_*i*=1_^2^(*x*_*i*_ − *a*_*ij*_)^6^))^−1^	2	[-65, 65]	1
*F*_15_(*x*) = ∑_*i*=1_^11^ [*a*_*i*_ − *x*_1_(*b*_*i*_^2^ − *b*_*i*_*x*_2_)/*b*_*i*_^2^ + *b*_*i*_*x*_3_ + *x*_4_]^2^	4	[-5, 5]	0.00030
*F*_16_(*x*) = 4*x*_1_^2^ − 2.1*x*_1_^2^ + 1/3*x*_1_^6^ + *x*_1_*x*_2_ − 4*x*_2_^2^ + 4*x*_2_^4^	2	[-5, 5]	-1.0316
*F*_17_(*x*) = (*x*_2_ − (5.1/4*π*^2^)*x*_1_^2^ + (5/*π*)*x*_1_ − 6)^2^ + 10(1 − 1/8*π*)cos*x*_1_ + 10	2	[-5, 5]	0.398
*F*_18_(*x*) = [1 + (*x*_1_ + *x*_2_ + 1)^2^(19 − 14*x*_1_ + 3*x*_1_^2^ − 14*x*_2_ + 6*x*_1_*x*_2_ + 3*x*_2_^2^)] × [30 + (2*x*_1_ − 3*x*_2_)^2^ × (18 − 32*x*_1_ + 12*x*_1_^2^ + 48*x*_2_ − 36*x*_1_*x*_2_ + 27*x*_2_^2^)]	2	[-2, 2]	3
*F*_19_(*x*) = −∑_*i*=1_^4^*c*_*i*_exp(−∑_*j*=1_^3^*a*_*ij*_(*x*_*j*_ − *p*_*ij*_])^2^)	3	[1, 3]	-3.86
*F*_20_(*x*) = −∑_*i*=1_^4^*c*_*i*_exp(−∑_*j*=1_^6^*a*_*ij*_(*x*_*j*_ − *p*_*ij*_])^2^)	6	[0, 1]	-3.32
*F*_21_(*x*) = −∑_*i*=1_^5^[(*X* − *a*_*i*_)(*X* − *a*_*i*_)^*T*^ + *c*_*i*_]^−1^	4	[0, 10]	-10.1532
*F*_22_(*x*) = −∑_*i*=1_^7^[(*X* − *a*_*i*_)(*X* − *a*_*i*_)^*T*^ + *c*_*i*_]^−1^	4	[0, 10]	-10.4028
*F*_23_(*x*) = −∑_*i*=1_^10^[(*X* − *a*_*i*_)(*X* − *a*_*i*_)^*T*^ + *c*_*i*_]^−1^	4	[0, 10]	-10.5363

The article "Boosting Slime Mould Algorithm for High-Dimensional Gene Data Mining: Diversity Analysis and Feature Selection" was published in 2022. Journal: Comput Math Methods Med.

**Table 4:** Descriptions of CEC2014 functions (search range: [−100, 100]D).

Function	Class	Functions	Optimum
F24	Hybrid	Hybrid 5: *N* = 5	2100
F25		Hybrid 6: *N* = 5	2200
F26	Composition	Composition 1: *N* = 5	2300
F27		Composition 2: *N* = 3	2400
F28		Composition 3: *N* = 3	2500
F29		Composition 4: *N* = 5	2600
F30		Composition 5: *N* = 5	2700
F31		Composition 6: *N* = 5	2800
F32		Composition 7: *N* = 3	2900
F33		Composition 8: *N* = 3	3000

**Table 5:** Experimental results of GLSMA, SMA, GSMA, and LSMA on 33 benchmark functions.

	F1		F2		F3	
	Avg	Std	Avg	Std	Avg	Std
GLSMA	*0.00E+00*	*0.00E+00*	*0.00E+00*	*0.00E+00*	*0.00E+00*	*0.00E+00*
SMA	0.00E+00	0.00E+00	0.00E+00	0.00E+00	0.00E+00	0.00E+00
GSMA	0.00E+00	0.00E+00	0.00E+00	0.00E+00	0.00E+00	0.00E+00
LSMA	0.00E+00	0.00E+00	0.00E+00	0.00E+00	0.00E+00	0.00E+00
	F4		F5		F6	
	Avg	Std	Avg	Std	Avg	Std
GLSMA	*0.00E+00*	*0.00E+00*	*1.29E-03*	*1.16E-03*	*7.00E-06*	*4.61E-06*
SMA	0.00E+00	0.00E+00	1.97E-03	1.01E-03	9.52E-06	4.12E-06
GSMA	0.00E+00	0.00E+00	1.96E-03	1.40E-03	1.32E-05	5.03E-06
LSMA	0.00E+00	0.00E+00	4.39E-03	2.62E-03	1.23E-05	5.56E-06
	F7		F8		F9	
	Avg	Std	Avg	Std	Avg	Std
GLSMA	*5.98E-06*	*5.13E-06*	-1.26E+04	1.07E-02	*0.00E+00*	*0.00E+00*
SMA	9.56E-06	8.00E-06	-1.26E+04	2.62E-04	0.00E+00	0.00E+00
GSMA	9.94E-06	9.90E-06	*-1.26E+04*	*2.32E-04*	0.00E+00	0.00E+00
LSMA	1.62E-05	1.41E-05	-1.27E+04	4.23E-04	0.00E+00	0.00E+00
	F10		F11		F12	
	Avg	Std	Avg	Std	Avg	Std
GLSMA	*8.88E-16*	*0.00E+00*	*0.00E+00*	*0.00E+00*	*2.35E-06*	*4.36E-06*
SMA	8.88E-16	0.00E+00	0.00E+00	0.00E+00	1.05E-05	1.00E-05
GSMA	8.88E-16	0.00E+00	0.00E+00	0.00E+00	8.42E-06	1.16E-05
LSMA	8.88E-16	0.00E+00	0.00E+00	0.00E+00	8.46E-06	8.61E-06
	F13		F14		F15	
	Avg	Std	Avg	Std	Avg	Std
GLSMA	*3.40E-06*	*2.79E-06*	*9.98E-01*	*4.51E-16*	3.12E-04	2.13E-05
SMA	6.59E-06	3.86E-06	9.98E-01	4.77E-16	*3.08E-04*	*1.89E-06*
GSMA	8.30E-06	5.62E-06	9.98E-01	5.49E-16	3.15E-04	3.67E-05
LSMA	8.12E-06	2.21E-06	9.98E-01	5.79E-16	3.21E-04	5.70E-05
	F16		F17		F18	
	Avg	Std	Avg	Std	Avg	Std
GLSMA	-1.03E+00	6.32E-14	*3.98E-01*	*7.20E-12*	*3.00E+00*	*1.04E-14*
SMA	-1.03E+00	1.21E-14	3.98E-01	1.32E-11	3.00E+00	1.16E-14
GSMA	*-1.03E+00*	*9.28E-15*	3.98E-01	1.14E-11	3.00E+00	1.21E-14
LSMA	-1.03E+00	1.31E-14	3.98E-01	2.58E-11	3.00E+00	1.03E-14
	F19		F20		F21	
	Avg	Std	Avg	Std	Avg	Std
GLSMA	-3.86E+00	6.18E-11	-3.24E+00	5.70E-02	-1.02E+01	1.27E-06
SMA	*-3.86E+00*	*4.13E-11*	-3.23E+00	4.84E-02	-1.02E+01	1.03E-06
GSMA	-3.86E+00	1.24E-10	-3.23E+00	4.84E-02	*-1.02E+01*	*9.16E-07*
LSMA	-3.86E+00	6.17E-11	*-3.21E+00*	*3.02E-02*	-1.02E+01	1.27E-06
	F22		F23		F24	
	Avg	Std	Avg	Std	Avg	Std
GLSMA	*-1.04E+01*	*9.50E-07*	*-1.05E+01*	*8.73E-07*	*1.05E+05*	*8.26E+04*
SMA	-1.04E+01	1.15E-06	-1.05E+01	1.06E-06	1.50E+05	4.96E+04
GSMA	-1.04E+01	1.56E-06	-1.05E+01	1.49E-06	1.16E+05	5.52E+04
LSMA	-1.04E+01	1.18E-06	-1.05E+01	1.44E-06	1.38E+05	6.74E+04
	F25		F26		F27	
	Avg	Std	Avg	Std	Avg	Std
GLSMA	*2.53E+03*	*1.78E+02*	*2.50E+03*	*0.00E+00*	*2.60E+03*	*0.00E+00*
SMA	2.70E+03	2.13E+02	2.50E+03	0.00E+00	2.60E+03	0.00E+00
GSMA	2.71E+03	1.75E+02	2.50E+03	0.00E+00	2.60E+03	0.00E+00
LSMA	2.65E+03	2.04E+02	2.50E+03	0.00E+00	2.60E+03	0.00E+00
	F28		F29		F30	
	Avg	Std	Avg	Std	Avg	Std
GLSMA	*2.70E+03*	*0.00E+00*	*2.70E+03*	*9.59E-02*	*2.90E+03*	*0.00E+00*
SMA	2.70E+03	0.00E+00	2.70E+03	1.42E-01	2.90E+03	0.00E+00
GSMA	2.70E+03	0.00E+00	2.70E+03	1.46E-01	2.90E+03	0.00E+00
LSMA	2.70E+03	0.00E+00	2.70E+03	1.21E-01	2.90E+03	0.00E+00
	F31		F32		F33	
	Avg	Std	Avg	Std	Avg	Std
GLSMA	*3.00E+03*	*0.00E+00*	*3.10E+03*	*0.00E+00*	*3.20E+03*	*0.00E+00*
SMA	3.00E+03	0.00E+00	4.11E+03	1.10E+03	5.38E+03	1.64E+03
GSMA	3.00E+03	0.00E+00	4.20E+03	1.12E+03	5.14E+03	1.67E+03
LSMA	3.00E+03	0.00E+00	3.89E+03	1.10E+03	5.67E+03	2.19E+03

The article "Boosting Slime Mould Algorithm for High-Dimensional Gene Data Mining: Diversity Analysis and Feature Selection" was published in 2022. Journal: Comput Math Methods Med.

**Table 6:** Wilcoxon signed-rank test results between GLSMA, SMA, GSMA, and LSMA.

Function	SMA	GMSA	LSMA	Function	SMA	GMSA	LSMA
F1	1.00E+00	1.00E+00	1.00E+00	F18	2.40E-01	5.15E-01	5.92E-01
F2	1.00E+00	1.0E+00	1.00E+00	F19	4.72E-02	8.61E-01	5.04E-01
F3	1.00E+00	1.00E+00	1.00E+00	F20	3.71E-01	3.19E-01	1.38E-03
F4	1.00E+00	1.00E+00	1.00E+00	F21	4.65E-01	7.81E-01	2.13E-01
F5	2.18E-02	1.75E-02	3.11E-05	F22	8.94E-01	8.98E-02	1.41E-01
F6	4.95E-02	4.53E-04	1.06E-04	F23	7.04E-01	2.18E-02	3.82E-01
F7	3.68E-02	1.41E-01	5.71E-04	F24	9.27E-03	6.58E-01	7.87E-02
F8	4.53E-04	1.38E-03	1.48E-03	F25	1.40E-02	4.90E-04	1.96E-02
F9	1.00E+00	1.00E+00	1.00E+00	F26	1.00E+00	1.00E+00	1.00E+00
F10	1.00E+00	1.00E+00	1.00E+00	F27	1.00E+00	1.00E+00	1.00E+00
F11	1.00E+00	1.00E+00	1.00E+00	F28	1.00E+00	1.00E+00	1.00E+00
F12	7.71E-04	8.73E-03	2.11E-03	F29	8.22E-02	1.78E-01	2.90E-01
F13	4.39E-03	7.71E-04	6.98E-06	F30	1.00E+00	1.00E+00	1000E+00
F14	5.08E-01	7.27E-01	5.081E-01	F31	1.00E+00	1.00E+00	1.00E+00
F15	1.11E-01	9.59E-01	7.66E-01	F32	6.10E-05	4.38E-04	6.10E-05
F16	3.37E-01	3.16E-01	1.32E-01	F33	5.96E-05	8.86E-05	1.32E-04
F17	3.49E-01	2.85E-02	2.99E-01	+/=/-	9/22/2	9/23/1	9/231

**Table 7:** Average ranking values using the Friedman test.

Algorithm	GLSMA	SMA	GSMA	LSMA
AVR	*1.454545*	1.878788	2.151515	2.30303
Rank	*1*	2	3	4

**Table 8:** Experimental results of GLSMA and seven original metaheuristic algorithms on 33 benchmark functions.

	F1		F2		F3	
	Avg	Std	Avg	Std	Avg	Std
GLSMA	*0.00E+00*	*0.00E+00*	*0.00E+00*	*0.00E+00*	*0.00E+00*	*0.00E+00*
PSO	1.03E+02	1.01E+01	4.58E+01	3.92E+00	1.94E+02	2.47E+01
WOA	0.00E+00	0.00E+00	0.00E+00	0.00E+00	4.18E+01	7.47E+01
GWO	0.00E+00	0.00E+00	0.00E+00	0.00E+00	2.37E-183	0.00E+00
SCA	2.04E-56	6.25E-56	1.69E-58	5.76E-58	5.41E+00	1.51E+01
FOA	2.50E-09	9.63E-12	2.74E-04	4.17E-07	7.88E-07	1.85E-09
DE	3.70E-159	1.03E-158	2.85E-94	4.33E-94	1.27E+03	5.02E+02
SSA	3.79E-09	9.30E-10	2.96E-01	5.45E-01	5.90E-08	1.81E-08
	F4		F5		F6	
	Avg	Std	Avg	Std	Avg	Std
GLSMA	*0.00E+00*	*0.00E+00*	1.24E-03	1.37E-03	6.31E-06	3.72E-06
PSO	3.82E+00	1.26E-01	*8.65E+04*	*2.0279E+04*	1.02E+02	1.14E+01
WOA	4.37E+00	1.06E+01	2.44E+01	7.73E-01	5.80E-06	2.37E-06
GWO	1.81E-152	4.50E-152	2.65E+01	8.77E-01	4.89E-01	2.88E-01
SCA	1.52E-02	6.23E-02	2.75E+01	6.24E-01	3.53E+00	2.92E-01
FOA	9.14E-06	1.46E-08	2.87E+01	1.09E-04	7.50E+00	3.59E-07
DE	3.17E-15	5.95E-15	3.29E+01	2.01E+01	*0.00E+00*	*0.00E+00*
SSA	1.92E-01	3.42E-01	4.59E+01	3.57E+01	3.81E-09	7.66E-10
	F7		F8		F9	
	Avg	Std	Avg	Std	Avg	Std
GLSMA	*7.45E-06*	*7.29E-06*	*-1.26E+04*	*1.27E-02*	*0.00E+00*	*0.00E+00*
PSO	1.11E+02	2.41E+01	-6.69E+03	8.24E+02	3.41E+02	1.52E+01
WOA	2.15E-04	2.53E-04	-1.24E+04	5.62E+02	0.00E+00	0.00E+00
GWO	6.44E-05	4.41E-05	-6.16E+03	6.56E+02	0.00E+00	0.00E+00
SCA	2.44E-03	2.59E-03	-4.42E+03	2.83E+02	1.18E-12	6.47E-12
FOA	3.15E-05	1.44E-05	-2.31E+02	1.13E+02	4.97E-07	1.73E-09
DE	2.39E-03	5.48E-04	-1.24E+04	1.29E+02	1.33E-01	3.44E-01
SSA	7.64E-03	3.24E-03	-7.76E+03	7.13E+02	6.91E+01	1.83E+01
	F10		F11		F12	
	Avg	Std	Avg	Std	Avg	Std
GLSMA	*8.88E-16*	*0.00E+00*	*0.00E+00*	*0.00E+00*	*1.16E-06*	*1.62E-06*
PSO	7.79E+00	3.02E-01	1.01E+00	9.86E-03	3.55E+00	3.93E-01
WOA	3.97E-15	2.59E-15	5.23E-04	2.86E-03	*9.31E-07*	*4.33E-07*
GWO	7.88E-15	6.49E-16	4.98E-04	1.90E-03	2.53E-02	1.77E-02
SCA	1.13E+01	9.36E+00	3.78E-09	2.07E-08	3.54E-01	1.30E-01
FOA	3.65E-05	4.17E-08	1.67E-10	6.21E-13	1.67E+00	6.05E-08
DE	7.53E-15	1.23E-15	0.00E+00	0.00E+00	1.57E-32	5.57E-48
SSA	1.78E+00	7.00E-01	1.28E-02	1.34E-02	9.54E-01	1.46E+00
	F13		F14		F15	
	Avg	Std	Avg	Std	Avg	Std
GLSMA	4.57E-06	2.70E-06	9.98E-01	4.76E-16	*3.08E-04*	*8.17E-07*
PSO	1.59E+01	1.70E+00	2.78E+00	2.17E+00	9.76E-04	5.57E-05
WOA	7.74E-04	2.78E-03	9.98E-01	1.10E-14	4.70E-04	3.12E-04
GWO	4.08E-01	1.69E-01	3.15E+00	3.56E+00	7.53E-03	1.29E-02
SCA	2.03E+00	1.27E-01	9.98E-01	6.09E-07	5.15E-04	3.78E-04
FOA	5.79E-01	7.79E-02	1.27E+01	1.04E-15	8.36E-04	2.74E-04
DE	*1.35E-32*	*5.57E-48*	*9.98E-01*	*0.00E+00*	3.72E-04	1.83E-04
SSA	3.60E-03	6.49E-03	9.98E-01	1.13E-16	7.38E-04	3.71E-04
	F16		F17		F18	
	Avg	Std	Avg	Std	Avg	Std
GLSMA	-1.03E+00	2.38E-14	3.98E-01	2.57E-12	*3.00E+00*	*1.16E-14*
PSO	-1.03E+00	9.52E-05	3.98E-01	6.35E-05	3.01E+00	7.37E-03
WOA	-1.03E+00	7.33E-15	3.98E-01	4.58E-10	3.00E+00	4.61E-08
GWO	-1.03E+00	2.82E-11	3.98E-01	4.01E-09	3.00E+00	8.51E-08
SCA	-1.03E+00	1.84E-06	3.98E-01	5.20E-05	3.00E+00	1.53E-07
FOA	-1.55E-01	1.29E-01	1.34E+00	8.72E-01	6.00E+02	1.89E-05
DE	-1.03E+00	6.78E-16	*3.98E-01*	*0.00E+00*	3.00E+00	2.03E-15
**SSA**	*-1.03E+00*	*6.14E-16*	3.98E-01	6.14E-16	3.00E+00	1.36E-14
	F19		F20		F21	
	Avg	Std	Avg	Std	Avg	Std
GLSMA	-3.86E+00	7.54E-11	-3.23E+00	4.84E-02	-1.02E+01	6.78E-07
PSO	-3.86E+00	2.82E-03	-2.92E+00	2.30E-01	-7.10E+00	1.54E+00
WOA	-3.86E+00	3.29E-03	-3.25E+00	8.23E-02	-1.02E+01	7.34E-07
GWO	-3.86E+00	2.00 E-03	-3.27E+00	7.29E-02	-9.98E+00	9.31E-01
SCA	-3.86E+00	3.107E-03	-2.98E+00	2.31E-01	-2.76E+00	2.52E+00
FOA	-3.62E+00	2.47E-01	-1.87E+00	4.40E-01	-3.68E+00	7.81E-01
DE	-3.86E+00	2.71E-15	*-3.3E+00*	*2.83E-04*	-9.90E+00	1.36E+00
SSA	*-3.86E+00*	*1.56E-15*	-3.23E+00	5.11E-02	*-1.02E+01*	*2.65E-12*
	F22		F23		F24	
	Avg	Std	Avg	Std	Avg	Std
GLSMA	-1.04E+01	9.95E-07	-1.05E+01	7.81E-07	1.19E+05	6.92E+04
PSO	-7.27E+00	1.19E+00	-7.50E+00	1.12E+00	9.22E+04	4.53E+04
WOA	-1.04E+01	2.57E-06	-1.05E+01	5.21E-07	1.40E+06	1.10E+06
GWO	-1.00E+01	1.35E+00	-1.05E+01	1.01E-06	1.02E+06	2.20E+06
SCA	-4.98E+00	3.34E+00	-4.66E+00	2.44E+00	1.29E+06	9.63E+05
FOA	-3.50E+00	8.81E-01	-3.40E+00	7.13E-01	8.34E+08	3.13E+08
DE	*-1.04E+01*	*1.81E-15*	*-1.05E+01*	*1.68E-15*	3.04E+05	1.59E+05
SSA	-9.70E+00	1.83E+00	-1.04E+01	9.79E-01	*5.96E+04*	*3.68E+04*
	F25		F26		F27	
	Avg	Std	Avg	Std	Avg	Std
GLSMA	2.64E+03	1.50E+02	*2.50E+03*	*0.00E+00*	*2.60E+03*	*0.00E+00*
PSO	2.90E+03	2.51E+02	2.62E+03	4.54E-01	2.63E+03	6.08E+00
WOA	2.97E+03	2.25E+02	2.63E+03	2.67E+01	2.61E+03	3.91E+00
GWO	2.59E+03	1.25E+02	2.64E+03	1.08E+01	2.60E+03	7.27E-04
SCA	2.99E+03	1.68E+02	2.66E+03	8.83E+00	2.60E+03	4.61E-02
FOA	1.25E+06	3.71E+05	2.50E+03	2.26E-06	2.60E+03	1.43E-05
DE	*2.40E+03*	*7.71E+01*	2.62E+03	1.39E-12	2.63E+03	3.42E+00
SSA	2.65E+03	2.00E+02	2.62E+03	1.77E-01	2.64E+03	8.96E+00
	F28		F29		F30	
	Avg	Std	Avg	Std	Avg	Std
GLSMA	*2.70E+03*	*0.00E+00*	2.70E+03	1.09E-01	*2.90E+03*	*0.00E+00*
PSO	2.71E+03	5.77E+00	2.78E+03	3.80E+01	3.45E+03	2.74E+02
WOA	2.72E+03	1.91E+01	2.70E+03	1.82E+01	3.72E+03	3.83E+02
GWO	2.71E+03	6.19E+00	2.76E+03	5.02E+01	3.37E+03	1.18E+02
SCA	2.73E+03	5.42E+00	2.70E+03	6.12E-01	3.44E+03	3.20E+02
FOA	2.70E+03	3.54E-08	2.80E+03	7.06E-11	2.90E+03	2.75E-07
DE	2.71E+03	1.04E+00	2.70E+03	4.42E-02	3.20E+03	8.08E+01
SSA	2.71E+03	4.09E+00	*2.70E+03*	*1.20E-01*	3.45E+03	1.46E+02
	F31		F32		F33	
	Avg	Std	Avg	Std	Avg	Std
GLSMA	*3.00E+03*	*0.00E+00*	*3.10E+03*	*0.00E+00*	*3.20E+03*	*0.00E+00*
PSO	7.19E+03	7.21E+02	8.87E+04	1.18E+05	1.55E+04	6.61E+03
WOA	5.04E+03	6.16E+02	4.55E+06	4.93E+06	7.94E+04	4.77E+04
GWO	3.97E+03	2.24E+02	1.87E+06	4.50E+06	5.28E+04	3.81E+04
SCA	4.83E+03	3.05E+02	1.04E+07	6.28E+06	2.19E+05	8.49E+04
FOA	3.00E+03	6.77E-07	4.65E+03	2.03E+00	3.31E+03	1.804E-01
DE	3.64E+03	2.41E+01	2.77E+04	1.16E+05	5.82E+03	9.58E+02
SSA	3.79E+03	8.08E+01	2.20E+06	5.20E+06	1.20E+04	4.50E+03

The article "Boosting Slime Mould Algorithm for High-Dimensional Gene Data Mining: Diversity Analysis and Feature Selection" was published in 2022. Journal: Comput Math Methods Med.

**Table 9:** Wilcoxon signed-rank test results between GLSMA and seven original metaheuristic algorithms.

Function	PSO	WOA	GWO	SCA	FOA	DE	SSA
F1	1.73E-06	1.00E+00	1.00E+00	1.73E-06	1.73E-06	1.73E-06	1.73E-06
F2	1.73E-06	1.00E+00	1.00E+00	1.73E-06	1.73E-06	1.73E-06	1.73E-06
F3	1.73E-06	1.73E-06	1.73E-06	1.73E-06	1.73E-06	1.73E-06	1.73E-06
F4	1.73E-06	1.73E-06	1.73E-06	1.73E-06	1.73E-06	1.73E-06	1.73E-06
F5	1.73E-06	1.73E-06	1.73E-06	1.73E-06	1.73E-06	1.73E-06	1.73E-06
F6	1.73E-06	7.50E-01	2.35E-06	1.73E-06	1.73E-06	1.73E-06	1.73E-06
F7	1.73E-06	1.73E-06	1.73E-06	1.73E-06	5.75E-06	1.73E-06	1.73E-06
F8	1.73E-06	4.99E-03	1.73E-06	1.73E-06	1.73E-06	1.36E-05	1.73E-06
F9	1.73E-06	1.00E+00	1.00E+00	1.00E+00	1.73E-06	1.25E-01	1.73E-06
F10	1.73E-06	4.15E-05	6.80E-08	1.73E-06	1.73E-06	1.96E-07	1.73E-06
F11	1.73E-06	1.00E+00	5.00E-01	1.00E+00	1.73E-06	1.00E+00	1.73E-06
F12	1.73E-06	5.72E-01	1.92E-06	1.73E-06	1.73E-06	1.73E-06	1.36E-05
F13	1.73E-06	1.73E-06	1.73E-06	1.73E-06	1.73E-06	1.73E-06	6.73E-01
F14	1.73E-06	6.13E-05	1.73E-06	1.73E-06	4.32E-08	4.32E-08	1.21E-07
F15	1.73E-06	4.45E-05	9.75E-01	1.73E-06	1.73E-06	7.97E-01	2.60E-05
F16	1.73E-06	1.55E-01	1.73E-06	1.73E-06	1.73E-06	1.14E-05	1.34E-04
F17	1.73E-06	3.16E-03	1.73E-06	1.73E-06	1.73E-06	1.73E-06	1.73E-06
F18	1.73E-06	1.73E-06	1.73E-06	1.73E-06	1.73E-06	1.53E-06	6.87E-01
F19	1.73E-06	1.73E-06	1.73E-06	1.73E-06	1.73E-06	1.73E-06	1.73E-06
F20	3.52E-06	8.13E-01	5.71E-02	1.73E-06	1.73E-06	1.92E-06	4.39E-03
F21	1.73E-06	1.36E-01	7.73E-03	1.73E-06	1.73E-06	3.11E-05	1.73E-06
F22	1.73E-06	4.11E-03	1.53E-01	1.73E-06	1.73E-06	1.73E-06	1.48E-02
F23	1.73E-06	4.99E-03	1.17E-02	1.73E-06	1.73E-06	1.73E-06	3.11E-05
F24	4.95E-02	2.60E-06	1.60E-04	1.73E-06	1.73E-06	2.88E-06	1.74E-04
F25	1.48E-04	6.98E-06	2.18E-02	2.13E-06	1.73E-06	1.36E-05	8.77E-01
F26	1.73E-06	2.56E-06	1.73E-06	1.73E-06	1.73E-06	4.32E-08	1.73E-06
F27	1.73E-06	1.73E-06	1.73E-06	1.73E-06	1.73E-06	1.73E-06	1.73E-06
F28	1.73E-06	2.93E-04	1.22E-05	1.73E-06	1.73E-06	1.73E-06	1.73E-06
F29	5.75E-06	9.84E-03	2.26E-03	1.73E-06	1.73E-06	3.18E-06	1.17E-02
F30	1.73E-06	1.73E-06	1.73E-06	1.73E-06	1.73E-06	1.73E-06	1.73E-06
F31	1.73E-06	1.73E-06	1.73E-06	1.73E-06	1.73E-06	1.73E-06	1.73E-06
F32	1.73E-06	1.72E-06	1.73E-06	1.73E-06	1.73E-06	1.73E-06	1.73E-06
F33	1.73E-06	1.73E-06	1.73E-06	1.73E-06	1.73E-06	1.73E-06	1.73E-06
+/=/-	32/0/1	22/91	25/7/1	31/2/0	33/0/0	17/3/13	21/3/9

The article "Boosting Slime Mould Algorithm for High-Dimensional Gene Data Mining: Diversity Analysis and Feature Selection" was published in 2022. Journal: Comput Math Methods Med.

**Table 10:** Average ranking values using the Friedman test.

Algorithm	GLSMA	PSO	WOA	GWO	SCA	FOA	DE	SSA
AVR	*2.328283*	6.591919	4.190404	4.187879	5.958081	5.80202	2.730303	4.211111
Rank	*1*	8	4	3	7	6	2	5

**Table 11:** Experimental results of GLSMA and eight advanced algorithms on 33 benchmark functions.

	F1		F2		F3	
	Avg	Std	Avg	Std	Avg	Std
GLSMA	*0.00E+00*	*0.00E+00*	*0.00E+00*	*0.00E+00*	*0.00E+00*	*0.00E+00*
MPEDE	2.37E-225	0.00E+00	1.61E-102	8.82E-102	1.61E-102	8.82E-102
LSHADE	1.22E-202	0.00E+00	1.46E-86	4.69E-86	1.46E-86	4.69E-86
ALCPSO	6.12E-186	0.00E+00	6.26E-05	2.21E-04	6.26E-05	2.21E-04
CLPSO	3.07E-34	2.84E-34	6.48E-21	2.80E-21	6.48E-21	2.80E-21
CMAES	1.93E-29	1.55E-30	5.24E-02	2.49E-01	5.24E-02	2.49E-01
BMWOA	4.41E-04	7.36E-04	6.11E-03	4.84E-03	6.11E-03	4.84E-03
CESCA	1.13E+03	7.79E+02	8.02E+00	1.94E+00	8.02E+00	1.94E+00
IGWO	0.00E+00	0.00E+00	3.84E-260	0.00E+00	3.84E-260	0.00E+00
	F4		F5		F6	
	Avg	Std	Avg	Std	Avg	Std
GLSMA	*0.00E+00*	*0.00E+00*	*1.69E-03*	*1.45E-03*	5.79E-06	3.48E-06
MPEDE	7.92E-06	1.05E-05	1.46E+00	1.95E+00	3.08E-33	4.05E-33
LSHADE	1.34E-04	1.91E-04	1.33E+00	1.91E+00	2.36E-33	4.10E-33
ALCPSO	3.92E-05	4.38E-05	3.59E+01	3.40E+01	2.33E-31	4.95E-31
CLPSO	1.32E+00	2.40E-01	4.82E-01	4.50E-01	*0.00E+00*	*0.00E+00*
CMAES	2.11E-15	1.18E-16	3.99E-01	1.22E+00	2.00E-29	1.64E-30
BMWOA	4.50E-03	4.85E-03	2.26E-02	5.96E-02	1.54E-03	3.03E-03
CESCA	2.00E+01	7.77E+00	2.88E+05	3.21E+05	1.25E+03	9.97E+02
IGWO	1.33E-38	7.27E-38	2.32E+01	2.03E-01	1.19E-05	4.26E-06
	F7		F8		F9	
	Avg	Std	Avg	Std	Avg	Std
GLSMA	*7.92E-06*	*5.81E-06*	*-1.26E+04*	*9.65E-03*	*0.00E+00*	*0.00E+00*
MPEDE	2.98E-03	1.02E-03	-1.19E+04	3.27E+02	7.67E+00	4.62E+00
LSHADE	6.16E-03	3.19E-03	-1.89E+03	2.65E+01	2.06E+00	3.60E+00
ALCPSO	8.49E-02	2.98E-02	-1.14E+04	2.88E+02	2.07E+01	7.79E+00
CLPSO	2.74E-03	7.42E-04	-1.26E+04	2.16E+01	0.00E+00	0.00E+00
CMAES	5.52E-02	1.56E-02	-7.13E+03	8.61E+02	2.30E+02	5.09E+01
BMWOA	1.17E-03	9.76E-04	-1.26E+04	1.03E-02	3.69E-04	6.17E-04
CESCA	4.93E-01	3.46E-01	-3.97E+03	2.51E+02	5.46E+01	1.26E+01
IGWO	3.76E-04	4.52E-04	-7.61E+03	6.63E+02	0.00E+00	0.00E+00
	F10		F11		F12	
	Avg	Std	Avg	Std	Avg	Std
GLSMA	*8.88E-16*	*0.00E+00*	*0.00E+00*	*0.00E+00*	1.68E-06	2.71E-06
MPEDE	1.60E+00	8.45E-01	2.02E-02	2.11E-02	1.77E-01	3.04E-01
LSHADE	3.38E-14	3.72E-15	1.43E-02	1.73E-02	7.08E-01	8.66E-01
ALCPSO	6.93E-01	8.23E-01	1.47E-02	1.73E-02	1.83E-02	3.50E-02
CLPSO	1.24E-14	2.59E-15	0.00E+00	0.00E+00	*1.57E-32*	*5.57E-48*
CMAES	1.94E+01	1.33E-01	1.23E-03	2.80E-03	1.07E-30	1.63E-31
BMWOA	2.11E-03	2.22E-03	9.96E-04	3.66E-03	7.11E-06	2.34E-05
CESCA	6.61E+00	1.41E+00	9.54E+00	5.47E+00	9.55E+04	1.70E+05
IGWO	4.91E-15	1.23E-15	0.00E+00	0.00E+00	1.09E-06	4.02E-07
	F13		F14		F15	
	Avg	Std	Avg	Std	Avg	Std
GLSMA	*3.08E-06*	*2.99E-06*	9.98E-01	5.77E-16	*3.09E-04*	*6.72E-06*
MPEDE	3.97E-03	6.58E-03	*9.98E-01*	*0.00E+00*	2.37E-03	6.10E-03
LSHADE	4.20E-01	1.14E+00	9.98E-01	0.00E+00	9.80E-04	3.64E-05
ALCPSO	7.73E-03	1.12E-02	9.98E-01	1.17E-16	3.69E-04	2.32E-04
CLPSO	1.35E-32	5.57E-48	9.98E-01	0.00E+00	5.50E-04	6.96E-05
CMAES	7.32E-04	2.79E-03	1.25E+01	6.58E+00	1.16E-02	2.06E-02
BMWOA	9.90E-05	1.76E-04	9.98E-01	3.13E-16	3.69E-04	2.32E-04
CESCA	7.14E+05	1.20E+06	2.87E+00	3.70E-01	4.38E-03	2.87E-03
IGWO	1.47E-02	3.56E-02	9.98E-01	3.01E-15	3.61E-04	2.05E-04
	F16		F17		F18	
	Avg	Std	Avg	Std	Avg	Std
GLSMA	-1.03E+00	2.81E-14	3.98E-01	4.35E-12	3.00E+00	1.26E-14
MPEDE	-1.03E+00	6.78E-16	*3.98E-01*	*0.00E+00*	3.00E+00	1.87E-15
LSHADE	-1.03E+00	6.78E-16	3.98E-01	0.00E+00	3.00E+00	1.20E-15
ALCPSO	-1.03E+00	6.39E-16	3.98E-01	0.00E+00	3.00E+00	2.66E-15
CLPSO	-1.03E+00	6.65E-16	3.98E-01	1.15E-15	*3.00E+00*	*1.17E-15*
CMAES	-9.72E-01	2.07E-01	3.98E-01	0.00E+00	3.46E+01	1.53E+02
BMWOA	*-1.0E+00*	*4.54E-16*	3.98E-01	2.57E-13	3.00E+00	1.30E-14
CESCA	-1.03E+00	5.79E-03	8.44E-01	3.91E-01	3.06E+00	8.45E-02
IGWO	-1.03E+00	5.32E-13	3.98E-01	6.44E-11	3.00E+00	4.95E-14
	F19		F20		F21	
	Avg	Std	Avg	Std	Avg	Std
GLSMA	-3.86E+00	4.37E-11	-3.23E+00	4.84E-02	*-1.02E+01*	*1.22E-06*
MPEDE	-3.86E+00	2.71E-15	-3.27E+00	5.99E-02	-8.81E+00	2.53E+00
LSHADE	-3.86E+00	7.59E-11	-1.63E+00	1.65E+00	-8.81E+00	2.53E+00
ALCPSO	*-3.86E+00*	*2.63E-15*	-3.27E+00	5.92E-02	-8.63E+00	2.36E+00
CLPSO	-3.86E+00	2.71E-15	*-3.32E+00*	*1.21E-12*	-1.02E+01	1.53E-06
CMAES	-3.58E+00	8.73E-01	-3.30E+00	4.84E-02	-5.92E+00	3.77E+00
BMWOA	-3.86E+00	2.26E-14	-3.26E+00	6.05E-02	-1.02E+01	3.44E-11
CESCA	-3.53E+00	2.38E-01	-2.05E+00	4.88E-01	-8.77E-01	3.53E-01
IGWO	-3.86E+00	2.66E-09	-3.26E+00	6.05E-02	-9.31E+00	1.93E+00
	F22		F23		F24	
	Avg	Std	Avg	Std	Avg	Std
GLSMA	-1.04E+01	1.03E-06	-1.05E+01	1.23E-06	1.14E+05	8.22E+04
MPEDE	-9.10E+00	2.70E+00	-1.03E+01	1.48E+00	3.06E+03	4.43E+02
LSHADE	-9.93E+00	1.82E+00	-1.00E+01	1.89E+00	*2.80E+03*	*2.66E+02*
ALCPSO	-9.52E+00	2.00E+00	-10.00E+00	1.64E+00	1.32E+05	2.18E+05
CLPSO	-1.04E+01	1.24E-06	-1.05E+01	5.43E-10	8.77E+04	6.01E+04
CMAES	-5.70E+00	3.22E+00	-7.16E+00	3.75E+00	3.18E+03	3.38E+02
BMWOA	*-1.04E+01*	*3.50E-11*	*-1.05E+01*	*2.87E-11*	1.10E+06	1.12E+06
CESCA	-1.18E+00	4.67E-01	-1.31E+00	5.62E-01	3.40E+07	1.28E+07
IGWO	-9.70E+00	1.83E+00	-10.00E+00	1.64E+00	3.08E+05	2.48E+05
	F25		F26		F27	
	Avg	Std	Avg	Std	Avg	Std
GLSMA	2.54E+03	1.70E+02	*2.50E+03*	*0.00E+00*	*2.60E+03*	*0.00E+00*
MPEDE	2.54E+03	1.54E+02	2.62E+03	1.68E-12	2.64E+03	5.74E+00
LSHADE	2.45E+03	1.17E+02	2.62E+03	2.13E-12	2.64E+03	5.18E+00
ALCPSO	2.67E+03	1.68E+02	2.62E+03	2.26E-02	2.64E+03	6.89E+00
CLPSO	*2.42E+03*	*7.90E+01*	2.62E+03	3.14E-06	2.62E+03	7.39E+00
CMAES	2.54E+03	2.59E+02	2.62E+03	1.39E-12	2.661E+03	9.29E+01
BMWOA	3.00E+03	2.03E+02	2.50E+03	4.14E-01	2.60E+03	1.99E-01
CESCA	5.95E+03	1.75E+03	3.03E+03	1.03E+02	2.66E+03	1.74E+01
IGWO	2.55E+03	1.48E+02	2.62E+03	2.36E+00	2.60E+03	4.00E-03
	F28		F29		F30	
	Avg	Std	Avg	Std	Avg	Std
GLSMA	*2.70E+03*	*0.00E+00*	2.70E+03	1.27E-01	*2.90E+03*	*0.00E+00*
MPEDE	2.71E+03	5.13E+00	2.71E+03	3.04E+01	3.27E+03	1.51E+02
LSHADE	2.71E+03	3.82E+00	2.71E+03	3.45E+01	3.27E+03	9.40E+01
ALCPSO	2.71E+03	3.70E+00	2.76E+03	4.88E+01	3.47E+03	2.23E+02
CLPSO	2.71E+03	9.97E-01	*2.70E+03*	*6.83E-02*	3.13E+03	4.63E+01
CMAES	2.70E+03	2.03E+00	2.72E+03	5.81E+01	3.07E+03	3.98+01
BMWOA	2.70E+03	5.68E-03	2.71E+03	1.04E-01	2.90E+03	1.63E-01
CESCA	2.72E+03	8.91E+00	2.71E+03	1.44+00	3.98E+03	1.58E+02
IGWO	2.71E+03	2.75E+00	2.70E+03	1.71E-01	3.11E+03	4.03E+00
	F31		F32		F33	
	Avg	Std	Avg	Std	Avg	Std
GLSMA	*3.00E+03*	*0.00E+00*	*3.10E+03*	*0.00E+00*	*3.20E+03*	*0.00E+00*
MPEDE	4.00E+03	3.22E+02	1.72E+06	3.94E+06	5.62E+03	1.14E+03
LSHADE	3.77E+03	1.41E+02	3.71E+03	1.61E+02	5.56E+03	9.79E+02
ALCPSO	4.31E+03	4.70E+02	1.45E+06	4.41E+06	1.82E+04	2.92E+04
CLPSO	3.70E+03	5.81E+01	3.86E+03	1.14E+02	6.15E+03	8.22E+02
CMAES	6.49E+03	2.96E+03	3.67E+03	1.31E+02	5.23E+03	6.37E+02
BMWOA	3.00E+03	5.17E-01	6.28E+05	6.18E+05	6.17E+04	5.38E+04
CESCA	5.43E+03	2.83E+02	1.78E+07	3.48E+06	1.42E+06	2.43E+05
IGWO	3.86E+03	1.94E+02	7.34E+05	2.75E+06	2.69E+04	1.15E+04

The article "Boosting Slime Mould Algorithm for High-Dimensional Gene Data Mining: Diversity Analysis and Feature Selection" was published in 2022. Journal: Comput Math Methods Med.

**Table 12:** Wilcoxon signed-rank test results between GLSMA and eight advanced algorithms.

Function	MPEDE	LSHADE	ALCPSO	CLPSO	CMAES	BMWOA	CESCA	IGWO
F1	1.73E-06	1.73E-06	1.73E-06	1.73E-06	1.73E-06	1.73E-06	1.73E-06	1.00E+00
F2	1.73E-06	1.73E-06	1.73E-06	1.73E-06	1.73E-06	1.73E-06	1.73E-06	1.73E-06
F3	1.73E-06	1.73E-06	1.73E-06	1.73E-06	1.73E-06	1.73E-06	1.73E-06	1.73E-06
F4	1.73E-06	1.73E-06	1.73E-06	1.73E-06	1.73E-06	1.73E-06	1.73E-06	1.73E-06
F5	3.82E-01	6.44E-01	1.73E-06	1.73E-06	2.77E-03	1.59E-01	1.73E-06	1.73E-06
F6	1.73E-06	1.73E-06	1.73E-06	1.73E-06	1.73E-06	5.75E-06	1.73E-06	5.22E-06
F7	1.73E-06	1.73E-06	1.73E-06	1.73E-06	1.73E-06	1.73E-06	1.73E-06	1.73E-06
F8	1.73E-06	1.73E-06	1.73E-06	3.11E-05	1.73E-06	3.68E-02	1.73E-06	1.73E-06
F9	1.73E-06	4.92E-06	1.73E-06	1.00E+00	1.73E-06	1.73E-06	1.73E-06	1.00E+00
F10	1.71E-06	9.53E-07	1.44E-06	1.12E-06	1.73E-06	1.73E-06	1.73E-06	1.96E-07
F11	2.69E-05	8.79E-05	5.93E-05	1.00E+00	6.25E-02	1.73E-06	1.73E-06	1.00E+00
F12	4.72E-02	5.31E-05	3.82E-01	1.73E-06	1.73E-06	1.92E-01	1.73E-06	5.72E-01
F13	9.75E-01	3.71E-01	8.73E-03	1.73E-06	3.59E-04	9.71E-05	1.73E-06	1.73E-06
F14	1.21E-07	1.21E-07	1.21E-07	1.21E-07	1.90E-06	2.75E-04	1.73E-06	6.33E-06
F15	5.71E-02	1.73E-06	3.59E-04	1.73E-06	1.15-04	3.59E-04	1.73E-06	3.59E-04
F16	3.20E-06	3.20E-06	4.85E-06	3.20E-06	6.95E-04	7.32E-06	1.73E-06	6.98E-06
F17	1.73E-06	1.73E-06	1.73E-06	1.73E-06	1.73E-06	2.84E-05	1.73E-06	2.16E-05
F18	1.49E-06	1.54E-06	2.18E-06	1.54E-06	1.97E-02	1.12E-04	1.73E-06	6.62E-02
F19	1.73E-06	3.11E-05	1.73E-06	1.73E-06	2.77E-03	1.73E-06	1.73E-06	1.92E-06
F20	1.02E-05	1.38E-03	9.32E-06	1.73E-06	5.22E-06	1.80E-05	1.73E-06	5.30E-01
F21	3.71E-01	3.71E-01	9.75E-01	1.60E-04	3.61E-03	1.73E-06	1.73E-06	8.47E-06
F22	1.65E-01	3.59E-04	5.71E-02	3.11E-05	1.15E-04	1.73E-06	1.73E-06	6.34E-06
F23	3.11E-05	3.59E-04	2.77E-03	1.73E-06	4.72E-02	1.73E-06	1.73E-06	2.16E-05
F24	1.73E-06	1.73E-06	2.13E-01	1.36E-01	1.73E-06	1.73E-06	1.73E-06	1.48E-03
F25	9.92E-01	1.67E-02	3.33E-02	3.16E-03	6.58E-01	2.3534E-06	1.73E-06	8.77E-01
F26	4.32E-08	4.32E-08	1.73E-06	1.73E-06	4.32E-08	1.73E-06	1.73E-06	1.73E-06
F27	1.73E-06	1.73-06	1.73E-06	2.13E-06	1.73E-06	1.73E-06	1.73E-06	1.73E-06
F28	1.73E-06	1.73E-06	1.73E-06	1.73E-06	1.73E-06	1.73E-06	1.73E-06	1.73E-06
F29	9.78E-02	1.59E-01	8.92E-05	7.51E-05	8.97E-02	1.48E-02	1.73E-06	2.60E-05
F30	1.73E-06	1.73E-06	1.73E-06	1.73E-06	1.73E-06	1.73E-06	1.73E-06	1.73E-06
F31	1.73E-06	1.73E-06	1.73E-06	1.73E-06	1.73E-06	1.73E-06	1.73E-06	1.73E-06
F32	1.73E-06	1.73E-06	1.73E-06	1.73E-06	1.73E-06	1.73E-06	1.73E-06	1.73E-06
F33	1.73E-06	1.73E-06	1.73E-06	1.73E-06	1.73E-06	1.73E-06	1.73E-06	1.73E-06
+/=/-	18/7/8	21/4/8	22/4/7	16/3/14	25/3/5	21/2/10	33/0/0	26/7/0

**Table 13:** Average ranking values using the Friedman test.

Algorithm	GLSMA	MPEDE	LSHADE	ALCPSO	CLPSO	CMAES	BMWOA	CESCA	IGWO
AVR	*3.62929*	3.84293	4.20808	5.25202	3.93131	4.83384	5.16212	8.75455	5.38586
Rank	*1*	2	4	7	3	5	6	9	8

**Table 14:** Characteristics of gene expression datasets.

Datasets	Samples	Features	Categories
Colon	62	2000	2
SRBCT	83	2309	4
Leukemia	72	7131	2
Brain_Tumor1	90	5920	5
Brain_Tumor2	50	10368	4
CNS	60	7130	2
DLBCL	77	5470	2
Leukemia1	72	5328	3
Leukemia2	72	11226	3
Lung_Cancer	203	12601	3
Prostate_Tumor	102	10509	2
Tumors_9	60	5726	9
Tumors_11	174	12534	11
Tumors_14	308	15010	26

The article "Boosting Slime Mould Algorithm for High-Dimensional Gene Data Mining: Diversity Analysis and Feature Selection" was published in 2022. Journal: Comput Math Methods Med.

**Table 15:** Comparison between BGLSMA and other FS optimizers on average number of the selected features.

Datasets	Metrics	bGWO	BBA	BGSA	BPSO	bALO	BSSA	BSMA	BGLSMA
Colon	Std	20.7964	54.9142	26.5991	12.8966	18.8043	318.1085	17.0098	*0.52705*
	Avg	165.4	781.7	768.8	891.9	856.6	768.1	32	*1.5*
SRBCT	Std	12.3306	67.0439	18.7723	21.6972	21.4828	336.9647	24.8697	*6.1968*
	Avg	186.6	933	906.8	1029.1	998.2	978.9	34.5	*11.2*
Leukemia	Std	45.8786	186.7911	33.7377	22.1761	34.2379	1602.754	12.5526	*0.5164*
	Avg	793.2	2991.7	3119.7	3334	3269.3	2046.7	39.3	*1.4*
Brain_Tumor1	Std	52.7674	163.1894	36.7792	51.0565	60.6781	1004.231	73.4078	*7.5491*
	Avg	623.2	2393.1	2564.6	2771.1	2732.5	2164.1	88.6	*6.9*
Brain_Tumor2	Std	57.3682	129.1005	45.7117	57.4886	52.4006	1816.777	114.1627	*5.1251*
	Avg	1191	1191	1191	1191	1191	1191	1191	*1191*
CNS	Std	35.9365	367.5338	59.1534	53.6694	68.2541	1448.946	116.9699	*1.4757*
	Avg	863.9	2848.3	3202.7	3391.8	3340.2	2456.3	199.2	*2.2*
DLBCL	Std	20.1594	153.9154	40.0012	32.3934	21.6705	1104.873	13.0826	*1.0593*
	Avg	567.2	2231.2	2358.1	2545	2495.5	2102.2	28.6	*1.7*
Leukemia1	Std	31.8462	133.4618	33.8856	36.5345	25.776	1035.249	62.1035	*20.1*
	Avg	564.8	2150.6	2283.7	2477.1	2433.8	1785.5	70.8	*13.7*
Leukemia2	Std	85.2763	256.4667	67.8352	47.7568	53.6723	2515.541	61.4167	*3.8355*
	Avg	1253.6	4632.5	5042.5	5335.6	5279.6	2553	76.3	*4.6*
Lung_Cancer	Std	117.4218	256.5553	73.7741	51.4295	46.6363	2856.425	182.022	*22.5982*
	Avg	1548.9	5207.2	5766.8	6020.9	5957.5	4110.1	206.3	*34.3*
Prostate_Tumor	Std	56.0124	607.9035	107.2774	58.1687	63.221	2544.318	128.1768	*2.5927*
	Avg	1281.5	4093.7	4834	5058.4	4974.7	2748.4	171.8	*4.5*
Tumors_9	Std	38.0935	139.8954	104.17	53.1402	48.8599	692.926	274.6595	*50.4341*
	Avg	661	2320.6	2572.5	2701.9	2661.8	2570.3	374.4	*28.4*
Tumors_11	Std	97.3416	668.8177	117.447	77.4884	*76.3216*	2645.298	308.9831	1207.602
	Avg	1639.5	1639.5	1639.5	1639.5	*1639.5*	1639.5	1639.5	1639.5
Tumors_14	Std	80.6821	499.8572	120.4111	*57.0264*	77.2704	1516.641	1914.11	2399.334
	Avg	2271.6	2271.6	2271.6	*2271.6*	2271.6	2271.6	2271.6	2271.6
ARV		2.9286	4.9286	5.8571	8	6.9286	4.2857	2	*1.0714*
Rank		3	5	6	8	7	4	2	*1*

**Table 16:** Comparison between BGLSMA and other FS optimizers on average error rate.

Datasets	Metrics	bGWO	BBA	BGSA	BPSO	bALO	BSSA	BSMA	BGLSMA
Colon	Std	6.549E-02	2.097E-01	1.277E-01	1.241E-01	1.365E-01	1.236E-01	0.000E+00	*0.000E+00*
	Avg	3.095E-02	2.619E-01	1.929E-01	1.571E-01	1.619E-01	1.810E-01	0.000E+00	*0.000E+00*
SRBCT	Std	0.000E+00	1.416E-01	0.000E+00	0.000E+00	0.000E+00	0.000E+00	0.000E+00	*0.000E+00*
	Avg	0.000E+00	1.237E-01	0.000E+00	0.000E+00	0.000E+00	0.000E+00	0.000E+00	*0.000E+00*
Leukemia	Std	0.000E+00	6.942E-02	0.000E+00	0.000E+00	0.000E+00	0.000E+00	0.000E+00	*0.000E+00*
	Avg	0.000E+00	5.357E-02	0.000E+00	0.000E+00	0.000E+00	0.000E+00	0.000E+00	*0.000E+00*
Brain_Tumor1	Std	5.197E-02	9.735E-02	7.147E-02	5.520E-02	7.216E-02	5.636E-02	4.216E-02	*3.162E-02*
	Avg	3.222E-02	1.081E-01	6.222E-02	5.222E-02	4.222E-02	5.333E-02	2.000E-02	*1.000E-02*
Brain_Tumor2	Std	7.770E-02	1.775E-01	1.370E-01	9.088E-02	9.875E-02	1.012E-01	0.000E+00	*0.000E+00*
	Avg	3.667E-02	2.850E-01	7.667E-02	7.000E-02	5.929E-02	6.167E-02	0.000E+00	*0.000E+00*
CNS	Std	5.271E-02	2.084E-01	8.784E-02	1.760E-01	8.635E-02	8.988E-02	4.518E-02	*0.000E+00*
	Avg	1.667E-02	4.171E-01	8.333E-02	1.143E-01	5.333E-02	8.429E-02	1.429E-02	*0.000E+00*
DLBCL	Std	3.953E-02	8.996E-02	4.518E-02	4.518E-02	3.953E-02	0.000E+00	0.000E+00	*0.000E+00*
	Avg	1.250E-02	7.857E-02	1.429E-02	1.429E-02	1.250E-02	0.000E+00	0.000E+00	*0.000E+00*
Leukemia1	Std	0.000E+00	1.214E-01	0.000E+00	0.000E+00	0.000E+00	0.000E+00	0.000E+00	*0.000E+00*
	Avg	0.000E+00	7.143E-02	0.000E+00	0.000E+00	0.000E+00	0.000E+00	0.000E+00	*0.000E+00*
Leukemia2	Std	0.000E+00	9.989E-02	0.000E+00	3.953E-02	0.000E+00	6.023E-02	0.000E+00	*0.000E+00*
	Avg	0.000E+00	0.000E+00	0.000E+00	0.000E+00	0.000E+00	0.000E+00	0.000E+00	*0.000E+00*
Lung_Cancer	Std	2.385E-02	4.691E-02	2.491E-02	3.310E-02	2.587E-02	3.376E-02	3.012E-02	*1.664E-02*
	Avg	1.479E-02	6.862E-02	1.929E-02	1.883E-02	2.452E-02	1.952E-02	9.524E-03	*5.263E-03*
Prostate_Tumor	Std	5.750E-02	1.470E-01	9.661E-02	5.182E-02	6.654E-02	6.542E-02	6.650E-02	*0.000E+00*
	Avg	1.818E-02	1.818E-02	1.818E-02	1.818E-02	1.818E-02	1.818E-02	1.818E-02	*1.818E-02*
Tumors_9	Std	*0.000E+00*	2.171E-01	*0.000E+00*	1.125E-01	9.223E-02	1.265E-01	3.953E-02	7.027E-02
	Avg	*0.000E+00*	4.168E-01	*0.000E+00*	5.000E-02	5.417E-02	4.000E-02	1.250E-02	3.333E-02
Tumors_11	Std	*1.757E-02*	8.280E-02	3.749E-02	4.035E-02	3.412E-02	6.182E-02	5.476E-02	3.857E-02
	Avg	*5.556E-03*	5.556E-03	5.556E-03	5.556E-03	5.556E-03	5.556E-03	5.556E-03	5.556E-03
Tumors_14	Std	*5.974E-02*	8.847E-02	7.256E-02	5.155E-02	6.288E-02	7.715E-02	6.560E-02	3.950E-02
	Avg	*1.908E-01*	3.376E-01	2.339E-01	2.781E-01	2.669E-01	3.063E-01	2.736E-01	2.787E-01
ARV		2	8	3.5714	4.4286	3.7857	4.7143	2	1.7143
Rank		2	8	4	6	5	7	2	1

The article "Boosting Slime Mould Algorithm for High-Dimensional Gene Data Mining: Diversity Analysis and Feature Selection" was published in 2022. Journal: Comput Math Methods Med.

**Table 17:** Comparison between BGLSMA and other FS optimizers on average fitness.

Datasets	Metrics	bGWO	BBA	BGSA	BPSO	bALO	BSSA	BSMA	BGLSMA
Colon	Std	6.219E-02	1.416E-01	1.214E-01	1.179E-01	1.298E-01	1.177E-01	4.253E-04	*1.318E-05*
	Avg	3.354E-02	2.032E-01	2.024E-01	1.716E-01	1.752E-01	1.911E-01	8.000E-04	*3.750E-05*
SRBCT	Std	2.671E-04	3.431E-02	4.067E-04	4.700E-04	4.654E-04	7.300E-03	5.388E-04	*1.343E-04*
	Avg	4.043E-03	2.862E-02	1.965E-02	2.229E-02	2.163E-02	2.121E-02	7.474E-04	*2.426E-04*
Leukemia	Std	3.217E-04	2.016E-03	2.366E-04	1.555E-04	2.401E-04	1.124E-02	8.803E-05	*3.621E-06*
	Avg	5.562E-03	1.924E-02	2.188E-02	2.338E-02	2.293E-02	1.435E-02	2.756E-04	*9.818E-06*
Brain_Tumor1	Std	4.935E-02	6.543E-02	6.796E-02	5.232E-02	6.844E-02	4.909E-02	3.995E-02	*3.005E-02*
	Avg	3.588E-02	8.786E-02	8.077E-02	7.302E-02	6.319E-02	6.895E-02	1.975E-02	*9.558E-03*
Brain_Tumor2	Std	7.366E-02	1.106E-01	1.302E-01	8.625E-02	9.379E-02	9.388E-02	5.506E-04	*2.472E-05*
	Avg	4.058E-02	1.352E-01	9.527E-02	9.028E-02	7.990E-02	7.645E-02	7.345E-04	*2.122E-05*
CNS	Std	5.002E-02	2.023E-01	8.344E-02	1.670E-01	8.186E-02	9.031E-02	4.304E-02	*1.035E-05*
	Avg	2.189E-02	2.113E-01	1.016E-01	1.324E-01	7.409E-02	9.730E-02	1.497E-02	*1.543E-05*
DLBCL	Std	3.749E-02	4.246E-02	4.290E-02	4.277E-02	3.763E-02	1.010E-02	1.196E-04	*9.685E-06*
	Avg	1.706E-02	3.127E-02	3.513E-02	3.684E-02	3.469E-02	1.922E-02	2.615E-04	*1.554E-05*
Leukemia1	Std	2.989E-04	2.989E-04	2.989E-04	2.989E-04	2.989E-04	2.989E-04	2.989E-04	*2.989E-04*
	Avg	5.301E-03	4.443E-02	2.144E-02	2.325E-02	2.284E-02	1.676E-02	6.645E-04	*1.286E-04*
Leukemia2	Std	3.799E-04	3.799E-04	3.799E-04	3.799E-04	3.799E-04	3.799E-04	3.799E-04	*3.799E-04*
	Avg	5.584E-03	4.486E-02	2.246E-02	3.564E-02	2.352E-02	3.852E-02	3.399E-04	*2.049E-05*
Lung_Cancer	Std	2.298E-02	4.072E-02	2.363E-02	3.148E-02	2.459E-02	3.729E-02	2.851E-02	*1.579E-02*
	Avg	2.019E-02	6.019E-02	4.121E-02	4.178E-02	4.694E-02	3.486E-02	9.866E-03	*5.136E-03*
Prostate_Tumor	Std	5.479E-02	7.082E-02	9.162E-02	4.910E-02	6.320E-02	6.686E-02	6.357E-02	*1.234E-05*
	Avg	2.337E-02	2.337E-02	2.337E-02	2.337E-02	2.337E-02	2.337E-02	2.337E-02	*2.337E-02*
Tumors_9	Std	3.326E-04	1.828E-01	9.096E-04	1.071E-01	8.783E-02	1.214E-01	*3.912E-02*	6.714E-02
	Avg	5.772E-03	1.681E-01	2.246E-02	7.109E-02	7.470E-02	6.044E-02	*1.514E-02*	3.192E-02
Tumors_11	Std	*1.651E-02*	6.199E-02	3.563E-02	3.821E-02	3.251E-02	5.882E-02	5.134E-02	3.794E-02
	Avg	*1.182E-02*	1.030E-01	6.002E-02	6.892E-02	8.389E-02	8.022E-02	4.772E-02	4.175E-02
Tumors_14	Std	5.678E-02	8.676E-02	6.881E-02	4.890E-02	5.967E-02	7.255E-02	6.031E-02	*3.776E-02*
	Avg	1.888E-01	1.888E-01	1.888E-01	1.888E-01	1.888E-01	1.888E-01	1.888E-01	*1.888E-01*
ARV		2.5	7.5714	5.0714	6.3571	5.7143	5.0714	2.2143	*1.5*
Rank		3	8	4	7	6	4	2	*1*

**Table 18:** Comparison between BGLSMA and other FS optimizers on average computational time.

Datasets	Metrics	bGWO	BBA	BGSA	BPSO	bALO	BSSA	BSMA	BGLSMA
Colon	Std	2.5514	2.5514	2.5514	2.5514	*2.5514*	2.5514	2.5514	2.5514
	Avg	31.9062	30.4906	13.6746	8.584	*8.0335*	37.1659	70.1156	114.1263
SRBCT	Std	2.9138	2.9361	1.8018	0.91374	*0.8866*	3.2522	9.1156	16.0452
	Avg	34.0148	34.1434	17.2141	10.1891	*9.9331*	45.3289	79.6426	139.0788
Leukemia	Std	9.0416	8.7894	3.5903	1.6512	*1.437*	13.8392	27.5824	46.7772
	Avg	91.0773	86.08	41.7215	19.6962	*18.1027*	122.9642	235.5459	383.8539
Brain_Tumor1	Std	7.8949	7.2781	4.1147	1.5711	*2.0128*	11.921	15.8751	35.8179
	Avg	77.839	75.6561	37.1795	20.7058	*19.0823*	106.5918	204.8332	331.4628
Brain_Tumor2	Std	13.1514	10.441	6.5964	2.3475	*1.8691*	17.5793	39.2047	53.3446
	Avg	129.8032	116.4358	53.2582	20.6694	*18.4634*	170.6433	339.6091	519.5528
CNS	Std	8.7883	7.4052	4.2408	1.4574	*1.5028*	13.3078	28.6106	44.1968
	Avg	89.6331	86.575	38.5343	17.6038	*15.9767*	120.3373	235.2898	363.2358
DLBCL	Std	7.2489	6.5617	3.362	1.5989	*1.342*	10.6978	20.8082	28.7903
	Avg	71.175	67.8196	33.2668	16.5984	*16.1274*	95.6511	181.2594	299.2078
Leukemia1	Std	7.4559	7.4559	7.4559	7.4559	*7.4559*	7.4559	7.4559	7.4559
	Avg	70.1512	65.732	31.9728	15.5488	*14.9732*	92.9905	179.7238	284.7675
Leukemia2	Std	14.1082	13.8476	8.4149	3.1481	*3.1518*	20.2226	43.5071	64.6559
	Avg	139.8351	130.1774	62.3828	28.8214	*26.3602*	192.8016	369.2325	591.9679
Lung_Cancer	Std	20.2852	25.0081	17.671	9.2944	*3.67*	35.113	52.5769	136.7772
	Avg	186.6111	219.1699	141.8596	115.52	*114.9638*	281.4307	436.7065	893.1362
Prostate_Tumor	Std	14.2167	14.4316	6.592	4.633	*3.9045*	22.1621	26.0276	61.9174
	Avg	135.8685	130.3268	71.3971	37.1729	*36.0317*	187.0535	376.2129	565.8891
Tumors_9	Std	7.598	5.6978	3.1465	1.17	*1.4113*	10.018	18.957	26.6486
	Avg	72.981	73.0313	31.4313	15.3876	*14.656*	98.7644	228.8745	291.5208
Tumors_11	Std	19.6112	18.8848	19.1443	5.764	*9.1023*	37.9402	45.4794	98.5864
	Avg	179.912	193.265	121.7997	94.3676	*90.4458*	265.7033	519.6271	661.6608
Tumors_14	Std	32.6068	44.7828	15.9668	14.1586	*17.9125*	72.9596	45.6897	114.9044
	Avg	278.9632	368.5713	323.2499	287.037	*289.2344*	458.6548	714.792	835.4772
ARV		4.4286	4.3571	3.0714	2	*1.1429*	6	7	8
Rank		5	4	3	2	*1*	6	7	8

The article "Boosting Slime Mould Algorithm for High-Dimensional Gene Data Mining: Diversity Analysis and Feature Selection" was published in 2022. Journal: Comput Math Methods Med.

## Data Availability

The data involved in this study are all public data, which can be downloaded through public channels.

## References

[1] Zhang X., Wang D., Zhou Z., Ma Y. (2021). Robust low-rank tensor recovery with rectification and alignment. *IEEE Transactions on Pattern Analysis and Machine Intelligence*.

[2] Deng W., Zhao H., Zou L., Li G., Yang X., Wu D. (2017). A novel collaborative optimization algorithm in solving complex optimization problems. *Soft Computing*.

[3] Storn R. (2005). Designing nonstandard filters with differential evolution. *IEEE Signal Processing Magazine*.

[4] Kennedy J., Mendes R. (2006). Neighborhood topologies in fully informed and best-of-neighborhood particle swarms. *Ieee Transactions on Systems Man and Cybernetics Part C-Applications and Reviews*.

[5] Heidari A. A., Mirjalili S., Faris H., Aljarah I., Mafarja M., Chen H. (2019). Harris hawks optimization: algorithm and applications. *Future Generation Computer Systems-the International Journal of Escience*.

[6] Ahmadianfar I., Heidari A. A., Gandomi A. H., Chu X., Chen H. (2021). RUN beyond the metaphor: an efficient optimization algorithm based on Runge Kutta method. *Expert Systems with Applications*.

[7] Yang Y., Chen H., Heidari A. A., Gandomi A. H. (2021). Hunger games search: visions, conception, implementation, deep analysis, perspectives, and towards performance shifts. *Expert Systems with Applications*.

[8] Li S., Chen H., Wang M., Heidari A. A., Mirjalili S. (2020). Slime mould algorithm: a new method for stochastic optimization. *Future Generation Computer Systems-the International Journal of Escience*.

[9] Wang G. G., Deb S., Cui Z. H. (2019). Monarch butterfly optimization. *Neural Computing & Applications*.

[10] Wang G. G. (2018). Moth search algorithm: a bio-inspired metaheuristic algorithm for global optimization problems. *Memetic Computing*.

[11] Tu J., Chen H., Wang M., Gandomi A. H. (2021). The colony predation algorithm. *Journal of Bionic Engineering*.

[12] Ahmadianfar I., Heidari A. A., Noshadian S., Chen H., Gandomi A. H. (2022). INFO: an efficient optimization algorithm based on weighted mean of vectors. *Expert Systems with Applications*.

[13] Ye X., Liu W., Li H. (2021). Modified whale optimization algorithm for solar cell and PV module parameter identification. *Complexity*.

[14] Dong R., Chen H., Heidari A. A., Turabieh H., Mafarja M., Wang S. (2021). Boosted kernel search: framework, analysis and case studies on the economic emission dispatch problem. *Knowledge-Based Systems*.

[15] Hussien A. G., Heidari A. A., Ye X., Liang G., Chen H., Pan Z. (2022). Boosting whale optimization with evolution strategy and Gaussian random walks: an image segmentation method. *Engineering with Computers*.

[16] Yu H., Song J., Chen C. (2022). Image segmentation of leaf spot diseases on maize using multi-stage Cauchy- enabled grey wolf algorithm. *Engineering Applications of Artificial Intelligence*.

[17] Yu H., Cheng X., Chen C. (2022). Apple leaf disease recognition method with improved residual network. *Multimedia Tools and Applications*.

[18] Xia J., Wang Z., Yang D. (2022). Performance optimization of support vector machine with oppositional grasshopper optimization for acute appendicitis diagnosis. *Computers in Biology and Medicine*.

The article "Boosting Slime Mould Algorithm for High-Dimensional Gene Data Mining: Diversity Analysis and Feature Selection" was published in 2022. Journal: Comput Math Methods Med.

[19] Xia J., Yang D., Zhou H. (2022). Evolving kernel extreme learning machine for medical diagnosis via a disperse foraging sine cosine algorithm. *Computers in Biology and Medicine*.

[20] Han X., Han Y., Chen Q. (2021). Distributed Flow shop scheduling with sequence-dependent setup times using an improved iterated greedy algorithm. *Complex System Modeling and Simulation*.

[21] Gao D., Wang G.-G., Pedrycz W. (2020). Solving fuzzy job-shop scheduling problem using DE algorithm improved by a selection mechanism. *IEEE Transactions on Fuzzy Systems*.

[22] Wang G.-G., Gao D., Pedrycz W. (2022). Solving multi-objective fuzzy job-shop scheduling problem by a hybrid adaptive differential evolution algorithm. *IEEE Transactions on Industrial Informatics*.

[23] ling Chen H., Yang B., Jing Wang S., Wang G., Zhong Li H., Bin Liu W. (2014). Towards an optimal support vector machine classifier using a parallel particle swarm optimization strategy. *Applied Mathematics and Computation*.

[24] Deng W., Zhang X., Zhou Y. (2022). An enhanced fast non-dominated solution sorting genetic algorithm for multi- objective problems. *Information Sciences*.

[25] Hua Y., Liu Q., Hao K., Jin Y. (2021). A survey of evolutionary algorithms for multi-objective optimization problems with irregular Pareto fronts. *IEEE/CAA Journal of Automatica Sinica*.

[26] Yu H., Yuan K., Li W. (2021). Improved butterfly optimizer-configured extreme learning machine for fault diagnosis. *Complexity*.

[27] Hu K., Ye J., Fan E., Shen S., Huang L., Pi J. (2017). A novel object tracking algorithm by fusing color and depth information based on single valued neutrosophic cross-entropy. *Journal of Intelligent Fuzzy Systems*.

[28] Hu K., He W., Ye J., Zhao L., Peng H., Pi J. (2019). Online visual tracking of weighted multiple instance learning via neutrosophic similarity-based objectness estimation. *Symmetry*.

[29] Wu S.-H., Zhan Z.-H., Zhang J. (2021). SAFE: scale-adaptive fitness evaluation method for expensive optimization problems. *IEEE Transactions on Evolutionary Computation*.

[30] Li J.-Y., Zhan Z. H., Wang C., Jin H., Zhang J. (2020). Boosting data-driven evolutionary algorithm with localized data generation. *IEEE Transactions on Evolutionary Computation*.

[31] Li Q., Chen H., Huang H. (2017). An enhanced grey wolf optimization based feature selection wrapped kernel extreme learning machine for medical diagnosis. *Computational and Mathematical Methods in Medicine*.

[32] Cai Z., Gu J., Wen C. (2018). An intelligent Parkinson’s disease diagnostic system based on a chaotic bacterial foraging optimization enhanced fuzzy KNN approach. *Computational and Mathematical Methods in Medicine*.

The article "Boosting Slime Mould Algorithm for High-Dimensional Gene Data Mining: Diversity Analysis and Feature Selection" was published in 2022. Journal: Comput Math Methods Med.

[33] Zhao F., di S., Cao J., Tang J., Jonrinaldi (2021). A novel cooperative multi-stage hyper-heuristic for combination optimization problems. *Complex System Modeling and Simulation*.

[34] Hu J., Chen H., Heidari A. A. (2021). Orthogonal learning covariance matrix for defects of grey wolf optimizer: insights, balance, diversity, and feature selection. *Knowledge-Based Systems*.

[35] Hu J., Gui W., Heidari A. A. (2022). Dispersed foraging slime mould algorithm: continuous and binary variants for global optimization and wrapper-based feature selection. *Knowledge-Based Systems*.

[36] Chen H., Wang M., Zhao X. (2020). A multi-strategy enhanced sine cosine algorithm for global optimization and constrained practical engineering problems. *Applied Mathematics and Computation*.

[37] Yu H., Qiao S., Heidari A. A., Bi C., Chen H. (2022). Individual disturbance and attraction repulsion strategy enhanced seagull optimization for engineering design. *Mathematics*.

[38] He Z., Yen G. G., Ding J. (2021). Knee-based decision making and visualization in many-objective optimization. *IEEE Transactions on Evolutionary Computation*.

[39] He Z., Yen G. G., Lv J. (2020). Evolutionary multiobjective optimization with robustness enhancement. *IEEE Transactions on Evolutionary Computation*.

[40] Kouadri R., Slimani L., Bouktir T. (2020). Slime mould algorithm for practical optimal power flow solutions incorporating stochastic wind power and static var compensator device. *Electrical Engineering & Electromechanics*.

[41] Khunkitti S., Siritaratiwat A., Premrudeepreechacharn S. (2021). Multi-objective optimal power Flow problems based on slime mould algorithm. *Sustainability*.

[42] Jafari-Asl J., Ohadi S., Ben Seghier M. E., Trung N. T. (2021). Accurate structural reliability analysis using an improved line-sampling-method-based slime mold algorithm. *Asce-Asme Journal of Risk and Uncertainty in Engineering Systems Part a-Civil Engineering*.

[43] Izci D., Ekinci S. (2021). Comparative performance analysis of slime mould algorithm for efficient design of proportional-integral-derivative controller. *Electrica*.

[44] Houssein E. H., Mahdy M. A., Shebl D., Manzoor A., Sarkar R., Mohamed W. M. (2022). An efficient slime mould algorithm for solving multi-objective optimization problems. *Expert Systems with Applications*.

[45] Houssein E. H., Mahdy M. A., Blondin M. J., Shebl D., Mohamed W. M. (2021). Hybrid slime mould algorithm with adaptive guided differential evolution algorithm for combinatorial and global optimization problems. *Expert Systems with Applications*.

[46] Gupta J., Nijhawan P., Ganguli S. (2021). Optimal parameter estimation of PEM fuel cell using slime mould algorithm. *International Journal of Energy Research*.

The article "Boosting Slime Mould Algorithm for High-Dimensional Gene Data Mining: Diversity Analysis and Feature Selection" was published in 2022. Journal: Comput Math Methods Med.

[47] Elsayed S. K., Agwa A. M., El-Dabbah M. A., Elattar E. E. (2021). Slime mold optimizer for transformer parameters identification with experimental validation. *Intelligent Automation and Soft Computing*.

[48] Hassan M. H., Kamel S., Abualigah L., Eid A. (2021). Development and application of slime mould algorithm for optimal economic emission dispatch. *Expert Systems with Applications*.

[49] Jia H., Zhang W., Zheng R., Wang S., Leng X., Cao N. (2022). Ensemble mutation slime mould algorithm with restart mechanism for feature selection. *International Journal of Intelligent Systems*.

[50] Altay O. (2022). Chaotic slime mould optimization algorithm for global optimization. *Artificial Intelligence Review*.

[51] Abdel-Basset M., Chang V., Mohamed R. (2020). HSMA_WOA: a hybrid novel slime mould algorithm with whale optimization algorithm for tackling the image segmentation problem of chest X-ray images. *Applied Soft Computing*.

[52] Chauhan S., Vashishtha G., Kumar A. (2022). A symbiosis of arithmetic optimizer with slime mould algorithm for improving global optimization and conventional design problem. *Journal of Supercomputing*.

[53] Alcalá-Fdez J., Sanchez L., Garcia S. (2009). KEEL: a software tool to assess evolutionary algorithms for data mining problems. *Soft Computing*.

[54] Mirjalili S., Lewis A. (2016). The whale optimization algorithm. *Advances in Engineering Software*.

[55] Mirjalili S., Mirjalili S., Lewis A. (2014). Grey wolf optimizer. *Advances in Engineering Software*.

[56] Mirjalili S. (2016). SCA: a sine cosine algorithm for solving optimization problems. *Knowledge-Based Systems*.

[57] Pan W.-T. (2012). A new fruit fly optimization algorithm: taking the financial distress model as an example. *Knowledge-Based Systems*.

[58] Mirjalili S., Gandomi A. H., Mirjalili S. Z., Saremi S., Faris H., Mirjalili S. M. (2017). Salp swarm algorithm: a bio-inspired optimizer for engineering design problems. *Advances in Engineering Software*.

[59] Wu G., Mallipeddi R., Suganthan P. N., Wang R., Chen H. (2016). Differential evolution with multi-population based ensemble of mutation strategies. *Information Sciences*.

[60] Piotrowski A. (2018). L-SHADE optimization algorithms with population-wide inertia. *Information Sciences*.

[61] Chen W., Zhang J., Lin Y. (2013). Particle swarm optimization with an aging leader and challengers. *IEEE Transactions on Evolutionary Computation*.

[62] Liang J., Qin A. K., Suganthan P. N., Baskar S. (2006). Comprehensive learning particle swarm optimizer for global optimization of multimodal functions. *IEEE Transactions on Evolutionary Computation*.

The article "Boosting Slime Mould Algorithm for High-Dimensional Gene Data Mining: Diversity Analysis and Feature Selection" was published in 2022. Journal: Comput Math Methods Med.

[63] Hansen N., Lozan J. A., Larrañaga P., Inza I., Bengoetxea E. (2006). The CMA Evolution Strategy: A Comparing Review. *Towards a New Evolutionary Computation: Advances in the Estimation of Distribution Algorithms*.

[64] Heidari A., Aljarah I., Faris H., Chen H., Luo J., Mirjalili S. (2020). An enhanced associative learning-based exploratory whale optimizer for global optimization. *Neural Computing & Applications*.

[65] Lin A., Wu Q., Heidari A. A. (2019). Predicting intentions of students for master programs using a chaos-induced sine cosine-based fuzzy K-nearest neighbor classifier. *Ieee Access*.

[66] Cai Z., Gu J., Luo J. (2019). Evolving an optimal kernel extreme learning machine by using an enhanced grey wolf optimization strategy. *Expert Systems with Applications*.

[67] Jadhav S., He H., Jenkins K. (2018). Information gain directed genetic algorithm wrapper feature selection for credit rating. *Applied Soft Computing*.

[68] Emary E., Zawba H., Hassanien A. (2016). Binary grey wolf optimization approaches for feature selection. *Neurocomputing*.

[69] Mirjalili S., Mirjalili S., Yang X. (2014). Binary bat algorithm. *Neural Computing & Applications*.

[70] Rashedi E., Nezamabadi-pour H., Saryazdi S. (2010). BGSA: binary gravitational search algorithm. *Natural Computing*.

[71] Mirjalili S., Lewis A. (2013). S-shaped versus V-shaped transfer functions for binary particle swarm optimization. *Swarm and Evolutionary Computation*.

[72] Emary E., Zawbaa H., Hassanien A. (2016). Binary ant lion approaches for feature selection. *Neurocomputing*.

[73] Reddy K., Panwar L. K., Panigrahi B. K., Kumar R. (2018). A new binary variant of sine-cosine algorithm: development and application to solve profit-based unit commitment problem. *Arabian Journal for Science and Engineering*.

[74] Qiu S., Zhao H., Jiang N. (2022). Multi-sensor information fusion based on machine learning for real applications in human activity recognition: state-of-the-art and research challenges. *Information Fusion*.

[75] Cao X., Sun X., Xu Z., Zeng B., Guan X. (2021). Hydrogen-based networked microgrids planning through two-stage stochastic programming with mixed-integer conic recourse. *IEEE Transactions on Automation Science and Engineering*.

[76] Guan Q., Chen Y., Wei Z. (2022). Medical image augmentation for lesion detection using a texture-constrained multichannel progressive GAN. *Computers in Biology and Medicine*.

[77] Hu Z., Wang J., Zhang C. (2022). Uncertainty modeling for multicenter autism spectrum disorder classification using Takagi–Sugeno–Kang fuzzy systems. *IEEE Transactions on Cognitive and Developmental Systems*.

The article "Boosting Slime Mould Algorithm for High-Dimensional Gene Data Mining: Diversity Analysis and Feature Selection" was published in 2022. Journal: Comput Math Methods Med.

[78] Su Y., Li S., Zheng C., Zhang X. (2020). A heuristic algorithm for identifying molecular signatures in cancer. *IEEE Transactions on Nanobioscience*.

[79] Li L., Gao Z., Wang Y. T. (2021). SCMFMDA: predicting microRNA-disease associations based on similarity constrained matrix factorization. *PLoS Computational Biology*.

[80] Yang Z., Ma J., Chen H., Zhang J., Chang Y. (2022). Context-aware attentive multi-level feature fusion for named entity recognition. *IEEE Transactions on Neural Networks and Learning Systems*.

[81] Wu Z., Li R., Zhou Z., Guo J., Jiang J., Su X. (2020). A user sensitive subject protection approach for book search service. *Journal of the Association for Information Science and Technology*.

[82] Wu Z., Shen S., Lian X., Su X., Chen E. (2020). A dummy-based user privacy protection approach for text information retrieval. *Knowledge-Based Systems*.

[83] Wu Z., Shen S., Zhou H., Li H., Lu C., Zou D. (2021). An effective approach for the protection of user commodity viewing privacy in e-commerce website. *Knowledge-Based Systems*.

[84] Wang D., Liang Y., Xu D., Feng X., Guan R. (2018). A content-based recommender system for computer science publications. *Knowledge-Based Systems*.

[85] Li J., Chen C., Chen H., Tong C. (2017). Towards context-aware social recommendation via individual trust. *Knowledge-Based Systems*.

[86] Li J., Lin J. (2020). A probability distribution detection based hybrid ensemble QoS prediction approach. *Information Sciences*.

[87] Li J., Zheng X. L., Chen S. T., Song W. W., Chen D. R. (2014). An efficient and reliable approach for quality-of-service-aware service composition. *Information Sciences*.

